The article "Dynamics of an Antitumour Model with Pulsed Radioimmunotherapy" was published in 2022. Journal: Comput Math Methods Med.

# Dynamics of an Antitumour Model with Pulsed Radioimmunotherapy

**DOI:** 10.1155/2022/4692772

**Published:** 2022-05-29

**Authors:** Gang Wang, Ming Yi, Sanyi Tang

**Affiliations:** ^1^School of Mathematics, Hunan Institute of Science and Technology, Yueyang 414006, China; ^2^School of Mathematics and Physics, China University of Geosciences, Wuhan 430074, China; ^3^School of Mathematics and Statistics, Shaanxi Normal University, Xi'an 710062, China

## Abstract

In this paper, an antitumour model for characterising radiotherapy and immunotherapy processes at different fixed times is proposed. The global attractiveness of the positive periodic solution for each corresponding subsystem is proved with the integral inequality technique. Then, based on the differentiability of the solutions with respect to the initial values, the eigenvalues of the Jacobian matrix at a fixed point corresponding to the tumour-free periodic solution are determined, resulting in a sufficient condition for local stability. The solutions to the ordinary differential equations are compared, the threshold condition for the global attractiveness of the tumour-free periodic solution is provided in terms of an indicator *R*_0_, and the permanence of a system with at least one tumour-present periodic solution is investigated. Furthermore, the effects of the death rate, effector cell injection dosage, therapeutic period, and effector cell activation rate on indicator *R*_0_ are determined through numerical simulations, and the results indicate that radioimmunotherapy is more effective than either radiotherapy or immunotherapy alone.

## 1. Introduction

Cancer is a major public health issue and the leading cause of death worldwide. According to the World Health Organization (WHO), there were nearly 10 million cancer-related deaths in 2020 [1]. The global cancer burden is expected to rise to nearly 21.4 million cases and 13.5 million deaths by 2030 [2]. Although numerous effective medical treatments against cancer have been developed, cancer treatment remains a challenging problem in neoteric medicine [3]. Host cells, or normal cells, should be kept above their minimum level throughout the entire body during cancer remission. As a result, modern techniques, such as surgery, chemotherapy, and radiotherapy, fail to destroy cancerous cells due to a lack of effective treatment strategies. In addition, chemotherapy harms cells in the bone marrow (myelosuppression), hair follicles (alopecia), and digestive tract (mucositis) under normal conditions. Therefore, chemotherapy depletes the immune system of the patient, leading to dangerous infections. Therefore, many patients suffer from the adverse effects of the treatment in addition to therapeutic resistance and cancer recurrence.

The article "Dynamics of an Antitumour Model with Pulsed Radioimmunotherapy" was published in 2022. Journal: Comput Math Methods Med.

Novel therapeutic strategies have been investigated, and immunotherapy has been recently approved for the treatment of various types of cancer [4]. Immunotherapy includes the use of antigen- and nonantigen-specific substances, such as cytokines, as well as adoptive cellular immunotherapy (ACI) [3]. Cytokines, such as IL-2 and IFN- *α*, are soluble proteins that mediate cell-to-cell communication [5]. During ACI, tissue cells are cultured to enhance and expand the immune system. ACI can be administered in two ways: (i) lymphokine-activated killer (LAK) cell therapy, in which cells are extracted from patients and cultured in vitro with high concentrations of IL-2 in peripheral blood leukocytes before being injected back into the cancer site; and (ii) tumour-infiltrating lymphocyte (TIL) therapy, in which cells are extracted from lymphocytes recovered from the patient with cancer and incubated with high concentrations of IL-2 before being injected back into the patient. The use of ACI slows or stops the spread of cancer cells to other parts of the body and helps the immune system become more effective by eliminating cancer cells.

Various mathematical models have been studied for cancer treatments with virotherapy, radiotherapy, chemotherapy, and immunotherapy [6–11]. Based on the inhibition model, Piantadosi model, and autostimulation model, Antonov et al. investigated impulsive tumour growth models to describe medical interventions during cancer treatments [12]. Sigal et al. modelled the effects of immunotherapy, specifically dendritic cell vaccines and T cell adoptive therapy, on tumour growth with and without chemotherapy [13]. The model demonstrated that chemotherapy increases tumorigenicity, whereas CSC-targeted immunotherapy tumorigenicity. Pratap proposed a model that describes the nonlinear dynamics between tumour cells, immune cells, and three forms of therapy: chemotherapy, immunotherapy, and radiotherapy [14]. The model was used to develop optimized combination therapy plans using optimal control theory. Feng and Navaratna demonstrated that the initial ratio between regulatory T cells and effector T cells impacts the tumour recurrence time and that the effectiveness of IL-2 use may reverse the immunotherapy outcome [15].

Dong et al. investigated the role of helper T cells in the tumour immune system and proposed the following model [16]:

(1) $$\begin{array}{c} \left\{\begin{array}{c} \frac{dx}{dt}=\alpha x\left(1-\beta x\right)-xy,\\ \begin{array}{c} \frac{dy}{dt}=\omega_{1}xy-\delta_{1}y+\rho yz,\\ \frac{dz}{dt}=\sigma_{2}+\omega_{2}xz-\delta_{2}z, \end{array} \end{array}\right. \end{array}$$

where *x*, *y*, and *z* represent the populations of tumour cells (TCs), effector cells (ECs), and helper T cells (HTCs), respectively. The first equation describes the rate of change in the TC population. Here, the logistic growth term *αx*(1 − *βx*) was chosen, where *α* is the maximal growth rate of the TC population, and 1/*β* is the carrying capacity of the TC biological environment. The second equation describes the rate of change in the EC population. ECs have an average lifespan of 1/*δ*_1_. *ω*_1_ is the EC stimulation rate by EC-lysed TC debris. *ρ* is the EC activation rate by the HTCs. The third equation describes the rate of change in the HTC population. *σ*_2_ is the birth rate of the HTCs produced in the bone marrow. HTCs have an average lifespan of 1/*δ*_2_. *ω*_2_ is the HTC stimulation rate in the presence of identified tumour antigens. To address the lack of biostability, Talkington et al. assumed that *ω*_1_ = 0 and introduced saturation into the tumour interactions [17]:

(2) $$\begin{array}{c} \left\{\begin{array}{c} \frac{dx}{d\tau }=\alpha x\left(1-\beta x\right)-y\frac{x}{x+\eta_{1}},\\ \frac{dy}{d\tau }=\sigma_{0}-\delta_{1}y+\rho yz,\\ \frac{dz}{d\tau }=\sigma_{2}-\delta_{2}z+\omega_{2}z\frac{x}{x+\eta_{3}}, \end{array}\right. \end{array}$$

where *σ*_0_ > 0 is the birth rate of the ECs, and *η*_1_ and *η*_3_ are half-saturation constants.

The article "Dynamics of an Antitumour Model with Pulsed Radioimmunotherapy" was published in 2022. Journal: Comput Math Methods Med.

As discussed above, radiotherapy is usually used in cancer treatment because it permanently damages the DNA of tumour cells, destroying these cells [18, 19]. While nearby healthy tissue cells can suffer temporary damage from this radiation, these cells can repair the DNA damage and continue to grow normally. Numerous studies have shown that radioimmunotherapy is more effective for inhibiting tumour growth than radiotherapy [4, 20]. Thus, compared to the continuous system models mentioned above, we introduce pulsed ACI and radiotherapy into system (2) and analyse the effect of the combined treatment [7, 21–23]. Our novel system is formulated as follows:

(3) $$\begin{array}{c} \left\{\begin{array}{c} \left.\begin{array}{c} \frac{dy}{dt}=-\delta_{1}y+\rho yz,\\ \frac{dz}{dt}=\sigma_{2}-\delta_{2}z+\omega_{2}z\frac{x}{x+\eta_{3}},\\ \frac{dx}{dt}=\alpha x\left(1-\beta x\right)-y\frac{x}{x+\eta_{1}}, \end{array}\right\}t\neq \left(n-1\right)T+lT,t\neq nT,\\ \left.\begin{array}{c} y\left(t^{+}\right)=\left(1-p_{E}\right)y\left(t\right),\\ z\left(t^{+}\right)=\left(1-p_{H}\right)z\left(t\right),\\ x\left(t^{+}\right)=\left(1-p_{T}\right)x\left(t\right), \end{array}\right\}t=\left(n-1\right)T+lT,\\ \left.\begin{array}{c} y\left(t^{+}\right)=y\left(t\right)+\sigma_{1},\\ z\left(t^{+}\right)=z\left(t\right),\\ x\left(t^{+}\right)=x\left(t\right), \end{array}\right\}t=nT, \end{array}\right. \end{array}$$

where *p*_*E*_, *p*_*H*_, and *p*_*T*_ denote the death rates of the ECs, HTCs, and TCs due to radiotherapy at time *t* = (*n* − 1)*T* + *lT*, respectively. Here, 0 < *p*_*E*_, *p*_*H*_ < *p*_*T*_, 0 < *l* < 1, and *T* > 0 are the therapeutic period. *σ*_1_ > 0 represents the dosage of infusing the ECs with antitumour activity at time *t* = *nT*.

The article "Dynamics of an Antitumour Model with Pulsed Radioimmunotherapy" was published in 2022. Journal: Comput Math Methods Med.

In this article, we study the effects of impulsive perturbations on the tumour-free solution of model (3) and the threshold values of its stability conditions. In addition, the mathematical criteria for the permanence of system (3) are investigated. Numerical simulations were carried out to validate our analytical results.

The article is organized as follows. In Section 2, for convenience, we present some definitions and lemmas. In Section 3, the local stability and global attractiveness of the tumour-free periodic solution are studied by means of the linearized Floquet stability and comparison techniques. Several additional technical computations that were used to establish the results presented in this section are deferred to see appendix. In Section 4, it is shown that once the threshold condition is satisfied, as well as certain other conditions, system (3) is permanent, with at least one tumour-present periodic solution. Numerical simulations that confirm our theoretical findings are discussed in Section 5 and Figures 1 and 2. Finally, a discussion of the theoretical and numerical results is provided.

## 2. Preliminaries

In this section, we introduce some definitions and preliminary lemmas that are useful for establishing our results.

**Definition 1 (see [24]).**

System (3) is said to be permanent if there are constants *m*, *M* > 0 (independent of the initial values) and a finite time *T*_0_ such that, for all solutions, (*y*(*t*), *z*(*t*), *x*(*t*)) with all initial values (*y*(0^+^), *z*(0^+^), *x*(0^+^)) > 0, *m* ≤ *y*(*t*), *z*(*t*) ≤ *M* and *m* ≤ *x*(*t*) ≤ *M* hold for all *T* ≥ *T*_0_. Here, *T*_0_ may depend on the initial value (*y*(0^+^), *z*(0^+^), *x*(0^+^)).

Similar to Lemma 1 in [21], we obtain that the solution of *d*Ψ(*t*)/*dt* = *χ*_1_(*t*)Ψ(*t*) + *χ*_2_(*t*) is

(4) $$\begin{array}{c} \Psi \left(t\right)=\Psi \left(t_{0}\right)e^{\int_{t_{0}}^{t}\chi_{1}\left(\tau \right)d\tau }+\int_{t_{0}}^{t}\chi_{2}\left(s\right)e^{-\int_{t}^{s}\chi_{1}\left(\tau \right)d\tau }ds. \end{array}$$

Thus, it follows that Ψ(*t*) ≥ 0 for Ψ(*t*_0_) ≥ 0, with *χ*_2_(*t*) ≥ 0 and *t* ≥ *t*_0_. Then, the following lemma is valid.

**Lemma 1 .**

The article "Dynamics of an Antitumour Model with Pulsed Radioimmunotherapy" was published in 2022. Journal: Comput Math Methods Med.

*R*_+_^3^ is a positively invariant region for system (3).

Let *x*(*t*) ≡ 0; then, system (3) can be reduced to the following system:

(5) $$\begin{array}{c} \left\{\begin{array}{c} \left.\begin{array}{c} \frac{dy}{dt}=-\delta_{1}y+\rho yz,\\ \frac{dz}{dt}=\sigma_{2}-\delta_{2}z, \end{array}\right\}t\neq \left(n-1\right)T+lT,t\neq nT,\\ \left.\begin{array}{c} y\left(t^{+}\right)=\left(1-p_{E}\right)y\left(t\right),\\ z\left(t^{+}\right)=\left(1-p_{H}\right)z\left(t\right), \end{array}\right\}t=\left(n-1\right)T+lT,\\ \left.\begin{array}{c} y\left(t^{+}\right)=y\left(t\right)+\sigma_{1},\\ z\left(t^{+}\right)=z\left(t\right), \end{array}\right\}t=nT. \end{array}\right. \end{array}$$

According to (5), we can obtain that

(6) $$\begin{array}{c} y\left(t\right)=\left\{\begin{array}{c} y\left(\left(n-1\right)T^{+}\right)e^{\int_{\left(n-1\right)T^{+}}^{t}\left(-\delta_{1}+\rho z\left(s\right)\right)ds},\\ \left(n-1\right)T<t\leq \left(n-1\right)T+lT,\\ y\left({\left(\left(n-1\right)T+lT\right)}^{+}\right)e^{\int_{{\left(\left(n-1\right)T+lT\right)}^{+}}^{t}\left(-\delta_{1}+\rho z\left(s\right)\right)ds},\\ \left(n-1\right)T+lT<t\leq nT, \end{array}\right. \end{array}$$

(7) $$\begin{array}{c} z\left(t\right)=\left\{\begin{array}{c} \frac{\sigma_{2}}{\delta_{2}}+\left(z\left(\left(n-1\right)T^{+}\right)-\frac{\sigma_{2}}{\delta_{2}}\right)e^{-\delta_{2}\left(t-\left(n-1\right)T\right)},\\ \left(n-1\right)T<t\leq \left(n-1\right)T+lT,\\ \frac{\sigma_{2}}{\delta_{2}}+\left(z\left({\left(\left(n-1\right)T+lT\right)}^{+}\right)-\frac{\sigma_{2}}{\delta_{2}}\right)e^{-\delta_{2}\left(t-\left(\left(n-1\right)T+lT\right)\right)},\\ \left(n-1\right)T+lT<t\leq nT. \end{array}\right. \end{array}$$

It is clear that

(8) $$\begin{array}{c} \left\{\begin{array}{c} y\left(nT^{+}\right)=\left(1-p_{E}\right)y\left(\left(n-1\right)T^{+}\right)e^{\int_{\left(n-1\right)T^{+}}^{nT}\left(-\delta_{1}+\rho z\left(t\right)\right)dt}+\sigma_{1},\\ z\left(nT^{+}\right)=\left[\left(1-e^{-\delta_{2}\left(1-l\right)T}\right)+\left(1-p_{H}\right)\left(e^{-\delta_{2}\left(1-l\right)T}-e^{-\delta_{2}T}\right)\right]\frac{\sigma_{2}}{\delta_{2}}+\left(1-p_{H}\right)e^{-\delta_{2}T}z\left(\left(n-1\right)T^{+}\right). \end{array}\right. \end{array}$$

Let

(9) $$\begin{array}{c} \left\{\begin{array}{c} y\left(nT^{+}\right)=y\left(\left(n-1\right)T^{+}\right),\\ z\left(nT^{+}\right)=z\left(\left(n-1\right)T^{+}\right); \end{array}\right. \end{array}$$

then, we have

(10) $$\begin{array}{c} \left\{\begin{array}{c} y\left(nT^{+}\right)=\frac{\sigma_{1}}{1-\left(1-p_{E}\right)e^{\int_{0^{+}}^{T}\left(-\delta_{1}+\rho z\left(t\right)\right)dt}},\\ z\left(nT^{+}\right)=\frac{\left[\left(1-e^{-\delta_{2}\left(1-l\right)T}\right)+\left(1-p_{H}\right)\left(e^{-\delta_{2}\left(1-l\right)T}-e^{-\delta_{2}T}\right)\right]\left(\sigma_{2}/\delta_{2}\right)}{1-\left(1-p_{H}\right)e^{-\delta_{2}T}}. \end{array}\right. \end{array}$$

Thus, when (15) is valid, system (5) has a unique positive periodic solution, which can be formulated as follows:

(11) $$\begin{array}{c} y^{*}\left(t\right)=\left\{\begin{array}{c} y^{*}\left(0^{+}\right)e^{\int_{\left(n-1\right)T^{+}}^{t}\left(-\delta_{1}+\rho z^{*}\left(s\right)\right)ds},\\ \left(n-1\right)T<t\leq \left(n-1\right)T+lT,\\ y^{*}\left(lT^{+}\right)e^{\int_{{\left(\left(n-1\right)T+lT\right)}^{+}}^{t}\left(-\delta_{1}+\rho z^{*}\left(s\right)\right)ds},\\ \left(n-1\right)T+lT<t\leq nT, \end{array}\right. \end{array}$$

(12) $$\begin{array}{c} z^{*}\left(t\right)=\left\{\begin{array}{c} \frac{\sigma_{2}}{\delta_{2}}+\left(z^{*}\left(0^{+}\right)-\frac{\sigma_{2}}{\delta_{2}}\right)e^{-\delta_{2}\left(t-\left(n-1\right)T\right)},\\ \left(n-1\right)T<t\leq \left(n-1\right)T+lT,\\ \frac{\sigma_{2}}{\delta_{2}}+\left(z^{*}\left(lT^{+}\right)-\frac{\sigma_{2}}{\delta_{2}}\right)e^{-\delta_{2}\left(t-\left(\left(n-1\right)T+lT\right)\right)},\\ \left(n-1\right)T+lT<t\leq nT, \end{array}\right. \end{array}$$

where

(13) $$\begin{array}{c} \left\{\begin{array}{c} y^{*}\left(0^{+}\right)=\frac{\sigma_{1}}{1-\left(1-p_{E}\right)e^{\int_{0^{+}}^{T}\left(-\delta_{1}+\rho z^{*}\left(t\right)\right)dt}},\\ y^{*}\left(lT^{+}\right)=\left(1-p_{E}\right)y^{*}\left(0^{+}\right)e^{\int_{0^{+}}^{lT}\left(-\delta_{1}+\rho z^{*}\left(t\right)\right)dt}, \end{array}\right. \end{array}$$

(14) $$\begin{array}{c} \left\{\begin{array}{c} z^{*}\left(0^{+}\right)=\frac{\left[\left(1-e^{-\delta_{2}\left(1-l\right)T}\right)+\left(1-p_{H}\right)\left(e^{-\delta_{2}\left(1-l\right)T}-e^{-\delta_{2}T}\right)\right]\left(\sigma_{2}/\delta_{2}\right)}{1-\left(1-p_{H}\right)e^{-\delta_{2}T}},\\ z^{*}\left(lT^{+}\right)=\left(1-p_{H}\right)\left(\frac{\sigma_{2}}{\delta_{2}}+\left(z^{*}\left(0^{+}\right)-\frac{\sigma_{2}}{\delta_{2}}\right)e^{-\delta_{2}lT}\right). \end{array}\right. \end{array}$$

Hence, we can obtain the following conclusion.

The article "Dynamics of an Antitumour Model with Pulsed Radioimmunotherapy" was published in 2022. Journal: Comput Math Methods Med.

**Lemma 2 .**

System (5) has a unique positive periodic solution (*y*^∗^(*t*), *z*^∗^(*t*)) if and only if

(15) $$\begin{array}{c} \left(1-p_{E}\right)e^{\int_{0^{+}}^{T}\left(-\delta_{1}+\rho z^{*}\left(t\right)\right)dt}<1, \end{array}$$

and, for every solution (*y*(*t*), *z*(*t*)) of (5), it follows that

(16) $$\begin{array}{c} \left\{\begin{array}{c} \underset{t⟶+\infty }{\lim}\left|y\left(t\right)-y^{*}\left(t\right)\right|=0,\\ \underset{t⟶+\infty }{\lim}\left|z\left(t\right)-z^{*}\left(t\right)\right|=0. \end{array}\right. \end{array}$$

**Proof**

It is easy to prove that $\underset{t⟶+\infty }{\lim}\left(z\left(t\right)-z^{*}\left(t\right)\right)=0$.

For an arbitrary *ε*^(1)^ > 0, we choose an *ε*_1_ > 0 that is sufficiently small such that

(17) $$\begin{array}{c} \left\{\begin{array}{c} C_{1}<1,\\ \frac{C_{2}e^{\rho \varepsilon_{1}T}}{1-C_{1}}<\frac{\varepsilon^{\left(1\right)}}{4e^{\rho \int_{0^{+}}^{T}z^{*}\left(t\right)dt}},\\ C_{3}<\frac{\varepsilon^{\left(1\right)}}{2}, \end{array}\right. \end{array}$$

where the first inequality in (17) is valid based on (15), and

(18) $$\begin{array}{c} \left\{\begin{array}{c} C_{1}=\left(1-p_{E}\right)e^{\int_{0^{+}}^{T}\left(-\delta_{1}+\rho \left(\varepsilon_{1}+z^{*}\left(t\right)\right)\right)dt},\\ C_{2}=\rho \varepsilon_{1}\left(\left(1-p_{E}\right)e^{\int_{0^{+}}^{T}\left(-\delta_{1}+\rho \left(\varepsilon_{1}+z^{*}\left(t\right)\right)\right)dt}\right.\times \int_{0^{+}}^{lT}y^{*}\left(t\right)e^{-\int_{0^{+}}^{t}\left(-\delta_{1}+\rho \left(\varepsilon_{1}+z^{*}\left(s\right)\right)\right)ds}dt+e^{\int_{lT^{+}}^{T}\left(-\delta_{1}+\rho \left(\varepsilon_{1}+z^{*}\left(t\right)\right)\right)dt}\left.\times \int_{lT^{+}}^{T}y^{*}\left(t\right)e^{-\int_{lT^{+}}^{t}\left(-\delta_{1}+\rho \left(\varepsilon_{1}+z^{*}\left(s\right)\right)\right)ds}dt\right),\\ C_{3}=\rho \varepsilon_{1}\left(e^{\rho \varepsilon_{1}T+\rho \int_{0^{+}}^{T}z^{*}\left(t\right)dt}\int_{0^{+}}^{lT}y^{*}\left(t\right)e^{\delta_{1}t}dt+\left.e^{\rho \varepsilon_{1}\left(1-l\right)T+\rho \int_{lT^{+}}^{T}z^{*}\left(t\right)dt}\int_{lT^{+}}^{T}y^{*}\left(t\right)e^{\delta_{1}\left(t-lT\right)}dt\right).\right. \end{array}\right. \end{array}$$

Without loss of generality, assume that

(19) $$\begin{array}{c} \left|z\left(t\right)-z^{*}\left(t\right)\right|<\varepsilon_{1}, \end{array}$$

for *t* ≥ 0.

When *t* ≠ (*n* − 1) + *lT*, *nT* and *y*(*t*) − *y*^∗^(*t*) ≠ 0, it follows from (5) and (19) that

(20) $$\begin{array}{c} \frac{d\left|y\left(t\right)-y^{*}\left(t\right)\right|}{dt}=\mathrm{sgn}\left(y\left(t\right)-y^{*}\left(t\right)\right)\times \left(-\delta_{1}\left(y\left(t\right)-y^{*}\left(t\right)\right)+\rho \left(y\left(t\right)z\left(t\right)-y^{*}\left(t\right)z^{*}\left(t\right)\right)\right)=-\delta_{1}\left|y\left(t\right)-y^{*}\left(t\right)\right|+\rho \mathrm{sgn}\left(y\left(t\right)-y^{*}\left(t\right)\right)\left[\left(y\left(t\right)-y^{*}\left(t\right)\right)z\left(t\right)+y^{*}\left(t\right)\left(z\left(t\right)-z^{*}\left(t\right)\right)\right]\leq \left(-\delta_{1}+\rho \left(\varepsilon_{1}+z^{*}\left(t\right)\right)\right)\left|y\left(t\right)-y^{*}\left(t\right)\right|+\rho \varepsilon_{1}y^{*}\left(t\right), \end{array}$$

which implies that

(21) $$\begin{array}{c} \frac{d}{dt}\left(\left|y\left(t\right)-y^{*}\left(t\right)\right|e^{-\int_{t_{0}}^{t}\left(-\delta_{1}+\rho \left(\varepsilon_{1}+z^{*}\left(s\right)\right)\right)ds}\right)\leq \rho \varepsilon_{1}y^{*}\left(t\right)e^{-\int_{t_{0}}^{t}\left(-\delta_{1}+\rho \left(\varepsilon_{1}+z^{*}\left(s\right)\right)\right)ds}. \end{array}$$

Integrating (21) from ((*n* − 1)*T*, *t*] or ((*n* − 1)*T* + *lT*, *t*] gives

(22) $$\begin{array}{c} \left|y\left(t\right)-y^{*}\left(t\right)\right|\leq \left\{\begin{array}{c} e^{\int_{\left(n-1\right)T^{+}}^{t}\left(-\delta_{1}+\rho \left(\varepsilon_{1}+z^{*}\left(s\right)\right)\right)ds}\left(\left|y\left(\left(n-1\right)T^{+}\right)-y^{*}\left(\left(n-1\right)T^{+}\right)\right|\left.+\int_{\left(n-1\right)T^{+}}^{t}\rho \varepsilon_{1}y^{*}\left(\tau \right)e^{-\int_{\left(n-1\right)T^{+}}^{\tau }\left(-\delta_{1}+\rho \left(\varepsilon_{1}+z^{*}\left(s\right)\right)\right)\;ds}d\tau \right),\right.\\ \left(n-1\right)T<t\leq \left(n-1\right)T+lT,\\ e^{\int_{{\left(\left(n-1\right)T+lT\right)}^{+}}^{t}\left(-\delta_{1}+\rho \left(\varepsilon_{1}+z^{*}\left(s\right)\right)\right)ds}\left(\left|y\left({\left(\left(n-1\right)T+lT\right)}^{+}\right)-y^{*}\left({\left(\left(n-1\right)T+lT\right)}^{+}\right)\right|+\int_{{\left(\left(n-1\right)T+lT\right)}^{+}}^{t}\rho \varepsilon_{1}y^{*}\left(\tau \right)e^{-\int_{{\left(\left(n-1\right)T+lT\right)}^{+}}^{\tau }\left(-\delta_{1}+\rho \left(\varepsilon_{1}+z^{*}\left(s\right)\right)\right)ds}d\tau \right),\\ \left(n-1\right)T+lT<t\leq nT. \end{array}\right. \end{array}$$

It should be noted that

(23) $$\begin{array}{c} \left\{\begin{array}{cc} \left|y\left(t^{+}\right)-y^{*}\left(t^{+}\right)\right|=\left(1-p_{E}\right)\left|y\left(t\right)-y^{*}\left(t\right)\right|, & t=\left(n-1\right)T+lT,\\ \left|y\left(t^{+}\right)-y^{*}\left(t^{+}\right)\right|=\left|y\left(t\right)-y^{*}\left(t\right)\right|, & t=nT. \end{array}\right. \end{array}$$

Then, it follows from (22) and (23) that

(24) $$\begin{array}{c} \left|y\left(nT^{+}\right)-y^{*}\left(nT^{+}\right)\right|\leq C_{1}\left|y\left(\left(n-1\right)T^{+}\right)-y^{*}\left(\left(n-1\right)T^{+}\right)\right|+C_{2}, \end{array}$$

which implies that

(25) $$\begin{array}{c} \left|y\left(nT^{+}\right)-y^{*}\left(nT^{+}\right)\right|\leq C_{1}^{n}\left(\left|y\left(0^{+}\right)-y^{*}\left(0^{+}\right)\right|-\frac{C_{2}}{1-C_{1}}\right)+\frac{C_{2}}{1-C_{1}}. \end{array}$$

Then, according to (25) and (17), there exists an *N*_1_ > 0 such that when *n* ≥ *N*_1_, it holds that

(26) $$\begin{array}{c} \left|y\left(nT^{+}\right)-y^{*}\left(nT^{+}\right)\right|<\frac{\varepsilon^{\left(1\right)}}{2e^{\rho \varepsilon_{1}T+\rho \int_{0^{+}}^{T}z^{*}\left(t\right)dt}}. \end{array}$$

Hence, when *t* ∈ ((*n* − 1)*T*, *nT*], where *n* − 1 ≥ *N*_1_, it follows from (22), (26), and (17) that

(27) $$\begin{array}{c} \left|y\left(t\right)-y^{*}\left(t\right)\right|\leq e^{\rho \varepsilon_{1}T+\rho \int_{0^{+}}^{T}z^{*}\left(t\right)dt}\left|y\left(\left(n-1\right)T^{+}\right)-y^{*}\left(\left(n-1\right)T^{+}\right)\right|+C_{3}<\varepsilon^{\left(1\right)}. \end{array}$$

Since *ε*^(1)^ > 0 is arbitrary, we conclude that $\underset{t⟶+\infty }{\lim}\left|y\left(t\right)-y^{*}\left(t\right)\right|=0$.

The article "Dynamics of an Antitumour Model with Pulsed Radioimmunotherapy" was published in 2022. Journal: Comput Math Methods Med.

This completes the proof.

Similarly, we arrive at the following conclusion.

**Lemma 3 .**

For every solution (*y*(*t*), *z*(*t*), *x*(*t*)) of system (3), there exist three positive constants *M*_*E*_, *M*_*H*_ > 0 and *M*_*T*_ > 0 such that

(28) $$\begin{array}{c} \left\{\begin{array}{c} y\left(t\right)\leq M_{E},\\ z\left(t\right)\leq M_{H},\\ x\left(t\right)\leq M_{T}, \end{array}\right. \end{array}$$

for sufficiently large *t* > 0, provided that

(29) $$\begin{array}{c} \left\{\begin{array}{c} \frac{\omega_{2}\left(1/\beta \right)}{\left(1/\beta \right)+\eta_{3}}<\delta_{2},\\ \left(1-p_{E}\right)e^{\int_{0^{+}}^{T}\left(-\delta_{1}+\rho {\overset{¯}{z}}_{0}\left(t\right)\right)dt}<1, \end{array}\right. \end{array}$$

where

(30) $$\begin{array}{c} {\overset{¯}{z}}_{0}\left(t\right)=\left\{\begin{array}{c} \frac{\sigma_{2}}{\delta_{2}-\omega_{2}\left(1/\beta \right)/\left(1/\beta \right)+\eta_{3}}+\left({\overset{¯}{z}}_{0}\left(0^{+}\right)-\frac{\sigma_{2}}{\delta_{2}-\omega_{2}\left(1/\beta \right)/\left(1/\beta \right)+\eta_{3}}\right)e^{-\left(\delta_{2}-\frac{\omega_{2}\left(1/\beta \right)}{\left(1/\beta \right)+\eta_{3}}\right)\left(t-\left(n-1\right)T\right)},\\ \left(n-1\right)T<t\leq \left(n-1\right)T+lT,\\ \frac{\sigma_{2}}{\delta_{2}-\omega_{2}\left(1/\beta \right)/\left(1/\beta \right)+\eta_{3}}+\left({\overset{¯}{z}}_{0}\left(lT^{+}\right)-\frac{\sigma_{2}}{\delta_{2}-\omega_{2}\left(1/\beta \right)/\left(1/\beta \right)+\eta_{3}}\right)e^{-\left(\delta_{2}-\frac{\omega_{2}\left(1/\beta \right)}{\left(1/\beta \right)+\eta_{3}}\right)\left(t-\left(\left(n-1\right)T+lT\right)\right)},\\ \left(n-1\right)T+lT<t\leq nT, \end{array}\right. \end{array}$$

with

(31) $$\begin{array}{c} \left\{\begin{array}{c} {\overset{¯}{z}}_{0}\left(0^{+}\right)=\frac{\left[\left(1-e^{-\left(\delta_{2}-\omega_{2}\left(1/\beta \right)/\left(1/\beta \right)+\eta_{3}\right)\left(1-l\right)T}\;\right)+\left(1-p_{H}\right)\left(e^{-\left(\delta_{2}-\omega_{2}\left(1/\beta \right)/\left(1/\beta \right)+\eta_{3}\right)\left(1-l\right)T}-e^{-\left(\delta_{2}-\omega_{2}\left(1/\beta \right)/\left(1/\beta \right)+\eta_{3}\right)T}\right)\right]\left(\sigma_{2}/\delta_{2}-\omega_{2}\left(1/\beta \right)/\left(1/\beta \right)+\eta_{3}\right)}{1-\left(1-p_{H}\right)e^{-\left(\delta_{2}-\omega_{2}\left(1/\beta \right)/\left(1/\beta \right)+\eta_{3}\right)T}},\\ {\overset{¯}{z}}_{0}\left(lT^{+}\right)=\left(1-p_{H}\right)\left(\frac{\sigma_{2}}{\delta_{2}-\omega_{2}\left(1/\beta \right)/\left(1/\beta \right)+\eta_{3}}+\left({\overset{¯}{z}}_{0}\left(0^{+}\right)-\frac{\sigma_{2}}{\delta_{2}-\omega_{2}\left(1/\beta \right)/\left(1/\beta \right)+\eta_{3}}\right)e^{-\left(\delta_{2}-\frac{\omega_{2}\left(1/\beta \right)}{\left(1/\beta \right)+\eta_{3}}\right)lT}\right). \end{array}\right. \end{array}$$

**Proof**

On the basis of (29), we choose an *ε*_*T*_ > 0 that is sufficiently small; then,

(32) $$\begin{array}{c} \left\{\begin{array}{c} \frac{\omega_{2}\left(\left(1/\beta \right)+\varepsilon_{T}\right)}{\left(\left(1/\beta \right)+\varepsilon_{T}\right)+\eta_{3}}<\delta_{2},\\ \left(1-p_{E}\right)e^{\int_{0^{+}}^{T}\left(-\delta_{1}+\rho {\overset{¯}{z}}^{*}\left(t\right)\right)dt}<1, \end{array}\right. \end{array}$$

where ${\overset{¯}{z}}^{*}\left(t\right)$ is defined in (36).

The article "Dynamics of an Antitumour Model with Pulsed Radioimmunotherapy" was published in 2022. Journal: Comput Math Methods Med.

According to Lemma 2 and (3), there exists a *t*_*T*_ > 0 such that when *t* > *t*_*T*_, it holds that

(33) $$\begin{array}{c} x\left(t\right)\leq \frac{1}{\beta }+\varepsilon_{T}≜M_{T}. \end{array}$$

Then, consider the following system:

(34) $$\begin{array}{c} \left\{\begin{array}{c} \left.\begin{array}{c} \frac{dy}{dt}=-\delta_{1}y+\rho yz,\\ \frac{dz}{dt}=\sigma_{2}-\left(\delta_{2}-\frac{\omega_{2}M_{T}}{M_{T}+\eta_{3}}\right)z, \end{array}\right\}t\neq \left(n-1\right)T+lT,t\neq nT,\\ \left.\begin{array}{c} y\left(t^{+}\right)=\left(1-p_{E}\right)y\left(t\right),\\ z\left(t^{+}\right)=\left(1-p_{H}\right)z\left(t\right), \end{array}\right\}t=\left(n-1\right)T+lT,\\ \left.\begin{array}{c} y\left(t^{+}\right)=y\left(t\right)+\sigma_{1},\\ z\left(t^{+}\right)=z\left(t\right), \end{array}\right\}t=nT, \end{array}\right. \end{array}$$

for *t* > *t*_*T*_. Similar to Lemma 3 it follows from (32) that

(35) $$\begin{array}{c} \left\{\begin{array}{c} \underset{t⟶+\infty }{\lim}\left|\overset{¯}{y}\left(t\right)-{\overset{¯}{y}}^{*}\left(t\right)\right|=0,\\ \underset{t⟶+\infty }{\lim}\left|\overset{¯}{z}\left(t\right)-{\overset{¯}{z}}^{*}\left(t\right)\right|=0, \end{array}\right. \end{array}$$

where $\left(\overset{¯}{y}\left(t\right),\overset{¯}{z}\left(t\right)\right)$ is a solution of (34), and

(36) $$\begin{array}{c} {\overset{¯}{z}}^{*}\left(t\right)=\left\{\begin{array}{c} \frac{\sigma_{2}}{\delta_{2}-\omega_{2}M_{T}/M_{T}+\eta_{3}}+\left({\overset{¯}{z}}^{*}\left(0^{+}\right)-\frac{\sigma_{2}}{\delta_{2}-\omega_{2}M_{T}/M_{T}+\eta_{3}}\right)e^{-\left(\delta_{2}-\frac{\omega_{2}M_{T}}{M_{T}+\eta_{3}}\right)\left(t-\left(n-1\right)T\right)},\\ \left(n-1\right)T<t\leq \left(n-1\right)T+lT,\\ \frac{\sigma_{2}}{\delta_{2}-\omega_{2}M_{T}/M_{T}+\eta_{3}}+\left({\overset{¯}{z}}^{*}\left(lT^{+}\right)-\frac{\sigma_{2}}{\delta_{2}-\omega_{2}M_{T}/M_{T}+\eta_{3}}\right)e^{-\left(\delta_{2}-\frac{\omega_{2}M_{T}}{M_{T}+\eta_{3}}\right)\left(t-\left(\left(n-1\right)T+lT\right)\right)},\\ \left(n-1\right)T+lT<t\leq nT, \end{array}\right. \end{array}$$

with

(37) $$\begin{array}{c} \left\{\begin{array}{c} {\overset{¯}{z}}^{*}\left(0^{+}\right)=\frac{\left[\left(1-e^{-\left(\delta_{2}-\omega_{2}M_{T}/M_{T}+\eta_{3}\right)\left(1-l\right)T}\right)+\left(1-p_{H}\right)\left(e^{-\left(\delta_{2}-\omega_{2}M_{T}/M_{T}+\eta_{3}\right)\left(1-l\right)T}-e^{-\left(\delta_{2}-\omega_{2}M_{T}/M_{T}+\eta_{3}\right)T}\right)\right]\left(\sigma_{2}/\delta_{2}-\omega_{2}M_{T}/M_{T}+\eta_{3}\right)}{1-\left(1-p_{H}\right)e^{-\left(\delta_{2}-\omega_{2}M_{T}/M_{T}+\eta_{3}\right)T}},\\ {\overset{¯}{z}}^{*}\left(lT^{+}\right)=\left(1-p_{H}\right)\left(\frac{\sigma_{2}}{\delta_{2}-\omega_{2}M_{T}/M_{T}+\eta_{3}}+\left({\overset{¯}{z}}^{*}\left(0^{+}\right)-\frac{\sigma_{2}}{\delta_{2}-\omega_{2}M_{T}/M_{T}+\eta_{3}}\right)e^{-\left(\delta_{2}-\frac{\omega_{2}M_{T}}{M_{T}+\eta_{3}}\right)lT}\right), \end{array}\right. \end{array}$$

and

(38) $$\begin{array}{c} {\overset{¯}{y}}^{*}\left(t\right)=\left\{\begin{array}{c} {\overset{¯}{y}}^{*}\left(0^{+}\right)e^{\int_{\left(n-1\right)T^{+}}^{t}\left(-\delta_{1}+\rho {\overset{¯}{z}}^{*}\left(s\right)\right)ds},\\ \left(n-1\right)T<t\leq \left(n-1\right)T+lT,\\ {\overset{¯}{y}}^{*}\left(lT^{+}\right)e^{\int_{{\left(\left(n-1\right)T+lT\right)}^{+}}^{t}\left(-\delta_{1}+\rho {\overset{¯}{z}}^{*}\left(s\right)\right)ds},\\ \left(n-1\right)T+lT<t\leq nT, \end{array}\right. \end{array}$$

with

(39) $$\begin{array}{c} \left\{\begin{array}{c} {\overset{¯}{y}}^{*}\left(0^{+}\right)=\frac{\sigma_{1}}{1-\left(1-p_{E}\right)e^{\int_{0^{+}}^{T}\left(-\delta_{1}+\rho {\overset{¯}{z}}^{*}\left(t\right)\right)dt}},\\ {\overset{¯}{y}}^{*}\left(lT^{+}\right)=\left(1-p_{E}\right){\overset{¯}{y}}^{*}\left(0^{+}\right)e^{\int_{0^{+}}^{lT}\left(-\delta_{1}+\rho {\overset{¯}{z}}^{*}\left(t\right)\right)dt}. \end{array}\right. \end{array}$$

Based on Lemma 2 and (3), it holds that $z\left(t\right)\leq \overset{¯}{z}\left(t\right)$ for *t* > *t*_*T*_; thus,

(40) $$\begin{array}{c} \left\{\begin{array}{cc} \frac{dy}{dt}\leq -\delta_{1}y+\rho y\overset{¯}{z}, & t\neq \left(n-1\right)T+lT,t\neq nT,\\ y\left(t^{+}\right)=\left(1-p_{E}\right)y\left(t\right), & t=\left(n-1\right)T+lT,\\ y\left(t^{+}\right)=y\left(t\right)+\sigma_{1}, & t=nT, \end{array}\right. \end{array}$$

for *t* > *t*_*T*_, which implies that $y\left(t\right)\leq \overset{¯}{y}\left(t\right)$ for *t* > *t*_*T*_. Thus, for arbitrary *ε*_*EH*_ > 0, there exists a *t*_*EH*_ > *t*_*T*_ such that when *t* > *t*_*EH*_, it holds that

(41) $$\begin{array}{c} \left\{\begin{array}{c} y\left(t\right)\leq \underset{t\in \left[0^{+},lT\right]\cup \left[lT^{+},T\right]}{\max}{\overset{¯}{y}}^{*}\left(t\right)+\varepsilon_{EH}≜M_{E},\\ z\left(t\right)\leq \underset{t\in \left[0^{+},lT\right]\cup \left[lT^{+},T\right]}{\max}{\overset{¯}{z}}^{*}\left(t\right)+\varepsilon_{EH}≜M_{H}. \end{array}\right. \end{array}$$

This completes the proof.

The article "Dynamics of an Antitumour Model with Pulsed Radioimmunotherapy" was published in 2022. Journal: Comput Math Methods Med.

## 3. The Stability of the Tumour-Free Periodic Solution

Let *Φ*(*t*; *t*_0_, *X*^0^) denote the solution of the first three equations of (3) for initial data *t* = *t*_0_ and *X*^0^ = (*y*^0^, *z*^0^, *x*^0^)^*T*^, as follows:

(42) $$\begin{array}{c} \Phi \left(t;t_{0},X^{0}\right)={\left(y\left(t;t_{0},X^{0}\right),z\left(t;t_{0},X^{0}\right),x\left(t;t_{0},X^{0}\right)\right)}^{T}. \end{array}$$

Additionally, we can define the mappings *I*_1_, *I*_2_ : *R*^3^⟶*R*^3^ as follows:

(43) $$\begin{array}{c} \left\{\begin{array}{c} I_{1}\left(y,z,x\right)=\left(\begin{array}{ccc} 1-p_{E} & 0 & 0\\ 0 & 1-p_{H} & 0\\ 0 & 0 & 1-p_{T} \end{array}\right)\left(\begin{array}{c} y\\ z\\ x \end{array}\right),\\ I_{2}\left(y,z,x\right)={\left(y,z,x\right)}^{T}+{\left(\sigma_{1},0,0\right)}^{T}, \end{array}\right. \end{array}$$

and the map Ψ : *R*^3^⟶*R*^3^ as

(44) $$\begin{array}{c} \Psi \left(X^{0}\right)=I_{2}\left(\Phi \left(\left(1-l\right)T,I_{1}\left(\Phi \left(lT,X^{0}\right)\right)\right)\right)={\left(y\left(T^{+};X^{0}\right),z\left(T^{+};X^{0}\right),x\left(T^{+};X^{0}\right)\right)}^{T}. \end{array}$$

**Theorem 1 .**

(i) The tumour-free periodic solution (*y*^∗^(*t*), *z*^∗^(*t*), 0) of system (3) is locally asymptotically stable provided that
  (45) $$\begin{array}{c} \;\left(1-p_{T}\right)e^{\alpha T-\int_{0}^{T}y^{*}\left(t\right)dt/\eta_{1}}<1. \end{array}$$
(ii) The tumour-free periodic solution (*y*^∗^(*t*), *z*^∗^(*t*), 0) of system (3) is globally attractive provided that
  (46) $$\begin{array}{c} R_{0}≜\left(1-p_{T}\right)e^{\alpha T-\int_{0^{+}}^{T}y^{*}\left(t\right)dt/\left(1/\beta \right)+\eta_{1}}<1. \end{array}$$

**Proof**

(1) According to (A.12), (A.13), (15), and (45), the three eigenvalues of the Jacobian matrix of map Ψ(*X*^0^) at point *X*_0_^∗^ = (*y*^∗^(0^+^), *z*^∗^(0^+^), 0) are

(47) $$\begin{array}{c} \left\{\begin{array}{c} \lambda_{1}=\left(1-p_{E}\right)e^{\int_{0^{+}}^{T}\left(-\delta_{1}+\rho z^{*}\left(t\right)\right)dt}<1,\\ \lambda_{2}=\left(1-p_{H}\right)e^{-\delta_{2}T}<1,\\ \lambda_{3}=\left(1-p_{T}\right)e^{\int_{0^{+}}^{T}\left(\alpha -\frac{y^{*}\left(t\right)}{\eta_{1}}\right)dt}<1, \end{array}\right. \end{array}$$

which implies that the tumour-free periodic solution (*y*^∗^(*t*), *z*^∗^(*t*), 0) is locally stable [25].

(2) Considering (46), we choose an $\varepsilon_{2}\in \left(0,\underset{t\in \left[0^{+},lT\right]\cup \left[lT^{+},T\right]}{\min}y^{*}\left(t\right)\right)$ such that

(48) $$\begin{array}{c} \zeta ≜\left(1-p_{T}\right)e^{\int_{0^{+}}^{T}\left(\alpha -\frac{y^{*}\left(t\right)-\varepsilon_{2}}{\left(\left(1/\beta \right)+\varepsilon_{2}\right)+\eta_{1}}\right)dt}<1. \end{array}$$

Let $\left(\hat{y}\left(t\right),\hat{z}\left(t\right)\right)$ denote the solution of (5). Then, according to Lemma 2 and (3), we have $z\left(t\right)\geq \hat{z}\left(t\right)$; thus,

(49) $$\begin{array}{c} \left\{\begin{array}{cc} \frac{dy}{dt}\geq -\delta_{1}y\left(t\right)+\rho y\left(t\right)\hat{z}\left(t\right), & t\neq \left(n-1\right)T+lT,t\neq nT,\\ y\left(t^{+}\right)=\left(1-p_{E}\right)y\left(t\right), & t=\left(n-1\right)T+lT,\\ y\left(t^{+}\right)=y\left(t\right)+\sigma_{1}, & t=nT, \end{array}\right. \end{array}$$

which implies that $y\left(t\right)\geq \hat{y}\left(t\right)$ [26]. Then, according to Lemmas 3 and 4, there exists a *t*_2_ > 0 such that

(50) $$\begin{array}{c} \left\{\begin{array}{c} y\left(t\right)\geq y^{*}\left(t\right)-\varepsilon_{2}>0,\\ x\left(t\right)\leq \frac{1}{\beta }+\varepsilon_{2}, \end{array}\right. \end{array}$$

for *t* > *t*_2_.

The article "Dynamics of an Antitumour Model with Pulsed Radioimmunotherapy" was published in 2022. Journal: Comput Math Methods Med.

Then, for *t* > *t*_2_, we have

(51) $$\begin{array}{c} \left\{\begin{array}{cc} \frac{dx}{dt}\leq x\left(\alpha -\frac{y^{*}\left(t\right)-\varepsilon_{2}}{\left(\left(1/\beta \right)+\varepsilon_{2}\right)+\eta_{1}}\right), & t\neq \left(n-1\right)T+lT,t\neq nT,\\ x\left(t^{+}\right)=\left(1-p_{T}\right)x\left(t\right), & t=\left(n-1\right)T+lT,\\ x\left(t^{+}\right)=x\left(t\right), & t=nT, \end{array}\right. \end{array}$$

which implies that

(52) $$\begin{array}{c} x\left(t\right)\leq \left\{\begin{array}{c} x\left(\left(n-1\right)T^{+}\right)e^{\int_{\left(n-1\right)T^{+}}^{t}\left(\alpha -\frac{y^{*}\left(t\right)-\varepsilon_{2}}{\left(\left(1/\beta \right)+\varepsilon_{2}\right)+\eta_{1}}\right)dt},\\ \left(n-1\right)T<t\leq \left(n-1\right)T+lT,\\ x\left({\left(\left(n-1\right)T+lT\right)}^{+}\right)e^{\int_{{\left(\left(n-1\right)T+lT\right)}^{+}}^{t}\left(\alpha -\frac{y^{*}\left(t\right)-\varepsilon_{2}}{\left(\left(1/\beta \right)+\varepsilon_{2}\right)+\eta_{1}}\right)dt},\\ \left(n-1\right)T+lT<t\leq nT. \end{array}\right. \end{array}$$

Furthermore, we have that

(53) $$\begin{array}{c} x\left(nT^{+}\right)\leq x\left(\left(n-1\right)T^{+}\right)\zeta . \end{array}$$

It follows from (48) and (53) that

(54) $$\begin{array}{c} \underset{n⟶\infty }{\lim}x\left(nT^{+}\right)=0. \end{array}$$

Moreover, it follows from (3) that

(55) $$\begin{array}{c} x\left(t\right)\leq x\left(\left(n-1\right)T^{+}\right)e^{\alpha T},\text{for }t\in \left(\left(n-1\right)T,nT\right]. \end{array}$$

Based on (54) and (55), we have $\underset{t⟶+\infty }{\lim}x\left(t\right)=0$.

The article "Dynamics of an Antitumour Model with Pulsed Radioimmunotherapy" was published in 2022. Journal: Comput Math Methods Med.

Similar to (50), we can prove that for arbitrary *ε*^(2)^ > 0, there exists a *t*^(2)^ > 0 such that

(56) $$\begin{array}{c} \left\{\begin{array}{c} y\left(t\right)>y^{*}\left(t\right)-\varepsilon^{\left(2\right)},\\ z\left(t\right)>z^{*}\left(t\right)-\varepsilon^{\left(2\right)}, \end{array}\right. \end{array}$$

for *t* > *t*^(2)^. In addition, we can choose an *ε*_3_ > 0 that is sufficiently small such that

(57) $$\begin{array}{c} \left\{\begin{array}{c} \frac{\omega_{2}\varepsilon_{3}}{\varepsilon_{3}+\eta_{3}}<\delta_{2},\\ \frac{\sigma_{2}\left(\omega_{2}\varepsilon_{3}/\varepsilon_{3}+\eta_{3}\right)}{\delta_{2}\left(\delta_{2}-\omega_{2}\varepsilon_{3}/\varepsilon_{3}+\eta_{3}\right)}+\left|\frac{{\overset{=}{z}}^{*}\left(0^{+}\right)}{z^{*}\left(0^{+}\right)}e^{\left(\omega_{2}\varepsilon_{3}/\varepsilon_{3}+\eta_{3}\right)lT}-1\right|z^{*}\left(0^{+}\right)<\frac{\varepsilon^{\left(2\right)}}{2},\\ \frac{\sigma_{2}\left(\omega_{2}\varepsilon_{3}/\varepsilon_{3}+\eta_{3}\right)}{\delta_{2}\left(\delta_{2}-\omega_{2}\varepsilon_{3}/\varepsilon_{3}+\eta_{3}\right)}+\left|\frac{{\overset{=}{z}}^{*}\left(lT^{+}\right)}{z^{*}\left(lT^{+}\right)}e^{\left(\omega_{2}\varepsilon_{3}/\varepsilon_{3}+\eta_{3}\right)\left(1-l\right)T}-1\right|z^{*}\left(lT^{+}\right)<\frac{\varepsilon^{\left(2\right)}}{2}, \end{array}\right. \end{array}$$

where ${\overset{=}{z}}^{*}\left(0^{+}\right)$ and ${\overset{=}{z}}^{*}\left(lT^{+}\right)$ are defined in (60).

Based on the fact that $\underset{t⟶+\infty }{\lim}x\left(t\right)=0$, there exists a *t*_3_ > *t*^(2)^ such that 0 < *x*(*t*) < *ε*_3_ for *t* > *t*_3_. Then, the following system is considered:

(58) $$\begin{array}{c} \left\{\begin{array}{cc} \frac{dz}{dt}=\sigma_{2}-\left(\delta_{2}-\frac{\omega_{2}\varepsilon_{3}}{\varepsilon_{3}+\eta_{3}}\right)z, & t\neq \left(n-1\right)T+lT,t\neq nT,\\ z\left(t^{+}\right)=\left(1-p_{H}\right)z\left(t\right), & t=\left(n-1\right)T+lT,\\ z\left(t^{+}\right)=z\left(t\right), & t=nT. \end{array}\right. \end{array}$$

For *t* > *t*_3_, we obtain the following positive periodic solution:

(59) $$\begin{array}{c} {\overset{=}{z}}^{*}\left(t\right)=\left\{\begin{array}{c} \frac{\sigma_{2}}{\delta_{2}-\omega_{2}\varepsilon_{3}/\varepsilon_{3}+\eta_{3}}+\left({\overset{=}{z}}^{*}\left(0^{+}\right)-\frac{\sigma_{2}}{\delta_{2}-\omega_{2}\varepsilon_{3}/\varepsilon_{3}+\eta_{3}}\right)e^{-\left(\delta_{2}-\frac{\omega_{2}\varepsilon_{3}}{\varepsilon_{3}+\eta_{3}}\right)\left(t-\left(n-1\right)T\right)},\\ \left(n-1\right)T<t\leq \left(n-1\right)T+lT,\\ \frac{\sigma_{2}}{\delta_{2}-\omega_{2}\varepsilon_{3}/\varepsilon_{3}+\eta_{3}}+\left({\overset{=}{z}}^{*}\left(lT^{+}\right)-\frac{\sigma_{2}}{\delta_{2}-\omega_{2}\varepsilon_{3}/\varepsilon_{3}+\eta_{3}}\right)e^{-\left(\delta_{2}-\frac{\omega_{2}\varepsilon_{3}}{\varepsilon_{3}+\eta_{3}}\right)\left(t-\left(\left(n-1\right)T+lT\right)\right)},\\ \left(n-1\right)T+lT<t\leq nT, \end{array}\right. \end{array}$$

with

(60) $$\begin{array}{c} \left\{\begin{array}{c} {\overset{=}{z}}^{*}\left(0^{+}\right)=\frac{\left[\left(1-e^{-\left(\delta_{2}-\omega_{2}\varepsilon_{3}/\varepsilon_{3}+\eta_{3}\right)\left(1-l\right)T}\right)+\left(1-p_{H}\right)\left(e^{-\left(\delta_{2}-\omega_{2}\varepsilon_{3}/\varepsilon_{3}+\eta_{3}\right)\left(1-l\right)T}-e^{-\left(\delta_{2}-\omega_{2}\varepsilon_{3}/\varepsilon_{3}+\eta_{3}\right)T}\right)\right]\left(\sigma_{2}/\delta_{2}-\omega_{2}\varepsilon_{3}/\varepsilon_{3}+\eta_{3}\right)}{1-\left(1-p_{H}\right)e^{-\left(\delta_{2}-\omega_{2}\varepsilon_{3}/\varepsilon_{3}+\eta_{3}\right)T}},\\ {\overset{=}{z}}^{*}\left(lT^{+}\right)=\left(1-p_{H}\right)\left(\frac{\sigma_{2}}{\delta_{2}-\omega_{2}\varepsilon_{3}/\varepsilon_{3}+\eta_{3}}+\left({\overset{=}{z}}^{*}\left(0^{+}\right)-\frac{\sigma_{2}}{\delta_{2}-\omega_{2}\varepsilon_{3}/\varepsilon_{3}+\eta_{3}}\right)e^{-\left(\delta_{2}-\frac{\omega_{2}\varepsilon_{3}}{\varepsilon_{3}+\eta_{3}}\right)lT}\right). \end{array}\right. \end{array}$$

Similar to Lemma 3, it follows from the first inequality of (57) that $\underset{n⟶\infty }{\lim}\left(\overset{=}{z}\left(t\right)-{\overset{=}{z}}^{*}\left(t\right)\right)=0$, where $\overset{=}{z}\left(t\right)$ is a solution of (58). Thus, there exists a *t*′_3_ > *t*_3_ such that

(61) $$\begin{array}{c} z\left(t\right)\leq \overset{=}{z}\left(t\right)<{\overset{=}{z}}^{*}\left(t\right)+\frac{\varepsilon^{\left(2\right)}}{2},\text{for }t>t\prime_{3}. \end{array}$$

When *t* > *t*′_3_, it follows from (59), (12), and (57) that

(62) $$\begin{array}{c} {\overset{=}{z}}^{*}\left(t\right)\leq z^{*}\left(t\right)+\frac{\sigma_{2}\left(\omega_{2}\varepsilon_{3}/\varepsilon_{3}+\eta_{3}\right)}{\delta_{2}\left(\delta_{2}-\omega_{2}\varepsilon_{3}/\varepsilon_{3}+\eta_{3}\right)}+\max\left\{\left|\frac{{\overset{=}{z}}^{*}\left(0^{+}\right)}{z^{*}\left(0^{+}\right)}e^{\left(\omega_{2}\varepsilon_{3}/\varepsilon_{3}+\eta_{3}\right)lT}-1\right|z^{*}\left(0^{+}\right),\left|\frac{{\overset{=}{z}}^{*}\left(lT^{+}\right)}{z^{*}\left(lT^{+}\right)}e^{\left(\omega_{2}\varepsilon_{3}/\varepsilon_{3}+\eta_{3}\right)\left(1-l\right)T}-1\right|z^{*}\left(lT^{+}\right)\right\}<z^{*}\left(t\right)+\frac{\varepsilon^{\left(2\right)}}{2}. \end{array}$$

Therefore, based on (61), (62), and (56), we can infer that

(63) $$\begin{array}{c} \left|z\left(t\right)-z^{*}\left(t\right)\right|<\varepsilon^{\left(2\right)},\text{for }t>t\prime_{3}. \end{array}$$

Since *ε*^(2)^ > 0 is arbitrary, we conclude that $\underset{t⟶+\infty }{\lim}\left(z\left(t\right)-z^{*}\left(t\right)\right)=0$.

The article "Dynamics of an Antitumour Model with Pulsed Radioimmunotherapy" was published in 2022. Journal: Comput Math Methods Med.

To prove that $\underset{t⟶+\infty }{\lim}\left(y\left(t\right)-y^{*}\left(t\right)\right)=0$, we choose an *ε*_4_ ∈ (0, *δ*_1_/*ρ*) such that

(64) $$\begin{array}{c} \left\{\begin{array}{c} \left(1-p_{E}\right)e^{\int_{0^{+}}^{T}\left(\left(\rho \varepsilon_{4}-\delta_{1}\right)+\rho z^{*}\left(t\right)\right)dt}<1,\\ \underset{t\in \left[0^{+},lT\right]}{\max}y^{*}\left(t\right)\left(\frac{{\overset{=}{y}}^{*}\left(0^{+}\right)}{y^{*}\left(0^{+}\right)}e^{\rho \varepsilon_{4}lT}-1\right)<\frac{\varepsilon^{\left(2\right)}}{2},\\ \underset{t\in \left[lT^{+},T\right]}{\max}y^{*}\left(t\right)\left(\frac{{\overset{=}{y}}^{*}\left(lT^{+}\right)e^{\rho \varepsilon_{4}T}}{y^{*}\left(lT^{+}\right)}-1\right)<\frac{\varepsilon^{\left(2\right)}}{2}, \end{array}\right. \end{array}$$

where the first inequality results from (15), and the expressions of ${\overset{=}{y}}^{*}\left(0^{+}\right)$ and ${\overset{=}{y}}^{**}\left(lT^{+}\right)$ are defined in (67).

Based on the fact that $\underset{t⟶+\infty }{\lim}\left(z\left(t\right)-z^{*}\left(t\right)\right)=0$, there exists a *t*_4_ > *t*^(2)^ such that *z*(*t*) < *z*^∗^(*t*) + *ε*_4_ for *t* > *t*_4_. Then, the following system is considered:

(65) $$\begin{array}{c} \left\{\begin{array}{cc} \frac{dy}{dt}=y\left(\left(\rho \varepsilon_{4}-\delta_{1}\right)+\rho z^{*}\left(t\right)\right), & t\neq \left(n-1\right)T+lT,t\neq nT,\\ y\left(t^{+}\right)=\left(1-p_{E}\right)y\left(t\right), & t=\left(n-1\right)T+lT,\\ y\left(t^{+}\right)=y\left(t\right)+\sigma_{1}, & t=nT. \end{array}\right. \end{array}$$

For *t* > *t*_4_, we obtain the following positive periodic solution:

(66) $$\begin{array}{c} {\overset{=}{y}}^{*}\left(t\right)=\left\{\begin{array}{c} {\overset{=}{y}}^{*}\left(0^{+}\right)e^{\int_{\left(n-1\right)T^{+}}^{t}\left(\left(\rho \varepsilon_{4}-\delta_{1}\right)+\rho z^{*}\left(s\right)\right)ds},\\ \left(n-1\right)T<t\leq \left(n-1\right)T+lT,\\ {\overset{=}{y}}^{*}\left(lT^{+}\right)e^{\int_{{\left(\left(n-1\right)T+lT\right)}^{+}}^{t}\left(\left(\rho \varepsilon_{4}-\delta_{1}\right)+\rho z^{*}\left(s\right)\right)ds},\\ \left(n-1\right)T+lT<t\leq nT, \end{array}\right. \end{array}$$

with

(67) $$\begin{array}{c} \left\{\begin{array}{c} {\overset{=}{y}}^{*}\left(0^{+}\right)=\frac{\sigma_{1}}{1-\left(1-p_{E}\right)e^{\int_{0^{+}}^{T}\left(\left(\rho \varepsilon_{4}-\delta_{1}\right)+\rho z^{*}\left(t\right)\right)dt}},\\ {\overset{=}{y}}^{*}\left(lT^{+}\right)=\left(1-p_{E}\right){\overset{=}{y}}^{*}\left(0^{+}\right)e^{\int_{0^{+}}^{lT}\left(\left(\rho \varepsilon_{4}-\delta_{1}\right)+\rho z^{*}\left(t\right)\right)dt}. \end{array}\right. \end{array}$$

According to (66), (11), and (64), when *t* > *t*_4_, it holds that

(68) $$\begin{array}{c} {\overset{=}{y}}^{*}\left(t\right)\leq y^{*}\left(t\right)+\max\left\{\underset{t\in \left[0^{+},lT\right]}{\max}y^{*}\left(t\right)\left(\frac{{\overset{=}{y}}^{*}\left(0^{+}\right)}{y^{*}\left(0^{+}\right)}e^{\rho \varepsilon_{4}lT}-1\right),\underset{t\in \left[lT^{+},T\right]}{\max}y^{*}\left(t\right)\left(\frac{{\overset{=}{y}}^{*}\left(lT^{+}\right)}{y^{*}\left(lT^{+}\right)}e^{\rho \varepsilon_{4}T}-1\right)\right\}<y^{*}\left(t\right)+\frac{\varepsilon^{\left(2\right)}}{2}. \end{array}$$

Similar to Lemma 3, we can prove that $\underset{t⟶+\infty }{\lim}\left(\overset{=}{y}\left(t\right)-{\overset{=}{y}}^{*}\left(t\right)\right)=0$, where $\overset{=}{y}\left(t\right)$ is a solution of (65). Thus, there exists a *t*′_4_ > *t*_4_ such that

(69) $$\begin{array}{c} y\left(t\right)\leq \overset{=}{y}\left(t\right)<y^{*}\left(t\right)+\varepsilon^{\left(2\right)},\text{for }t>t\prime_{4}. \end{array}$$

Therefore, based on (69) and (56), we can infer that

(70) $$\begin{array}{c} \left|y\left(t\right)-y^{*}\left(t\right)\right|<\varepsilon^{\left(2\right)},\text{for }t>t\prime_{4}. \end{array}$$

Since *ε*^(2)^ > 0 is arbitrary, we conclude that $\underset{t⟶+\infty }{\lim}\left(y\left(t\right)-y^{*}\left(t\right)\right)=0$.

The article "Dynamics of an Antitumour Model with Pulsed Radioimmunotherapy" was published in 2022. Journal: Comput Math Methods Med.

This completes the proof.

**Remark 1 .**

Since (45) can be inferred from (46), it follows from Theorem 5 that the tumour-free periodic solution (*y*^∗^(*t*), *z*^∗^(*t*), 0) of system (3) is globally asymptotically stable provided that (46) holds.

## 4. A Sufficient Condition for the Permanence of System (3)

In this section, we present some conditions for evaluating the permanence of system (46).

**Theorem 2 .**

System (3) is permanent with at least one positive periodic solution provided that (15), (29) and

(71) $$\begin{array}{c} \;\left(1-p_{T}\right)e^{\int_{0^{+}}^{T}\left(\alpha -\frac{y^{*}\left(t\right)}{\eta_{1}}\right)dt}>1 \end{array}$$

hold.

**Proof**

(29) implies that Lemma 4 holds; that is, there exist three positive constants *M*_*E*_, *M*_*H*_ > 0 and *M*_*T*_ > 0 such that *y*(*t*) < *M*_*E*_, *z*(*t*) < *M*_*H*_ and *x*(*t*) < *M*_*T*_ for all sufficiently large *t*. Without loss of generality, assume that *y*(*t*) < *M*_*E*_, *z*(*t*) < *M*_*H*_ and *x*(*t*) < *M*_*T*_ for *t* ≥ 0.

Moreover, (15) indicates that Lemma 3 holds. Thus, similar to (56), we can prove that

(72) $$\begin{array}{c} \left\{\begin{array}{c} y\left(t\right)>\underset{t\in \left[0^{+},lT\right]\cup \left[lT^{+},T\right]}{\min}y^{*}\left(t\right)-{\overset{¯}{\varepsilon }}_{E}≜m_{E},\\ z\left(t\right)>\underset{t\in \left[0^{+},lT\right]\cup \left[lT^{+},T\right]}{\min}z^{*}\left(t\right)-{\overset{¯}{\varepsilon }}_{H}≜m_{H}, \end{array}\right. \end{array}$$

for sufficiently large *t*, where

(73) $$\begin{array}{c} \left\{\begin{array}{c} {\overset{¯}{\varepsilon }}_{E}\in \left(0,\underset{t\in \left[0^{+},lT\right]\cup \left[lT^{+},T\right]}{\min}y^{*}\left(t\right)\right),\\ {\overset{¯}{\varepsilon }}_{H}\in \left(0,\underset{t\in \left[0^{+},lT\right]\cup \left[{lT}^{+},T\right]}{\min}z^{*}\left(t\right)\right). \end{array}\right. \end{array}$$

According to Definition 1, we only need to find *m*_*T*_ > 0 such that *x*(*t*) ≥ *m*_*T*_ for sufficiently large *t*. We can divide the process of determining *m*_*T*_ into two steps for convenience:

**Step 1 .**

According to (8) and (41), we can choose *m*_0_ > 0 and *ε*_5_ ∈ (0, *δ*_1_/*ρ*) such that

(74) $$\begin{array}{c} \left\{\begin{array}{c} \frac{\omega_{2}m_{0}}{m_{0}+\eta_{3}}<\delta_{2},\\ \left(1-p_{E}\right)e^{\int_{0^{+}}^{T}\left(\left(\rho \varepsilon_{5}-\delta_{1}\right)+\rho {\tilde{z}}^{*}\left(t\right)\right)dt}<1,\\ \eta \left(m_{0},\varepsilon_{5}\right)>1, \end{array}\right. \end{array}$$

where ${\tilde{z}}^{*}\left(t\right)$ and ${\tilde{y}}^{*}\left(t\right)$ are defined in (77) and (81), respectively, and

(75) $$\begin{array}{c} \eta \left(m_{0},\varepsilon_{5}\right)≜\left(1-p_{T}\right)e^{\int_{0^{+}}^{T}\left(\alpha -\alpha \beta m_{0}-\frac{{\tilde{y}}^{*}\left(t\right)+\varepsilon_{5}}{\eta_{1}}\right)dt}. \end{array}$$

Next, we consider the following system:

(76) $$\begin{array}{c} \left\{\begin{array}{cc} \frac{dz}{dt}=\sigma_{2}-\left(\delta_{2}-\frac{\omega_{2}m_{0}}{m_{0}+\eta_{3}}\right)z, & t\neq \left(n-1\right)T+lT,t\neq nT,\\ z\left(t^{+}\right)=\left(1-p_{H}\right)z\left(t\right), & t=\left(n-1\right)T+lT,\\ z\left(t^{+}\right)=z\left(t\right), & t=nT. \end{array}\right. \end{array}$$

Similar to Lemma 3, it follows from the first inequality of (74) that $\underset{t⟶+\infty }{\lim}\left(\tilde{z}\left(t\right)-{\tilde{z}}^{*}\left(t\right)\right)=0$, where $\tilde{z}\left(t\right)$ is the solution of (76), and

(77) $$\begin{array}{c} {\tilde{z}}^{*}\left(t\right)=\left\{\begin{array}{c} \frac{\sigma_{2}}{\delta_{2}-\omega_{2}m_{0}/m_{0}+\eta_{3}}+\left({\tilde{z}}^{*}\left(0^{+}\right)-\frac{\sigma_{2}}{\delta_{2}-\omega_{2}m_{0}/m_{0}+\eta_{3}}\right)e^{-\left(\delta_{2}-\frac{\omega_{2}m_{0}}{m_{0}+\eta_{3}}\right)\left(t-\left(n-1\right)T\right)},\\ \left(n-1\right)T<t\leq \left(n-1\right)T+lT,\\ \frac{\sigma_{2}}{\delta_{2}-\omega_{2}m_{0}/m_{0}+\eta_{3}}+\left({\tilde{z}}^{*}\left(lT^{+}\right)-\frac{\sigma_{2}}{\delta_{2}-\omega_{2}m_{0}/m_{0}+\eta_{3}}\right)e^{-\left(\delta_{2}-\frac{\omega_{2}m_{0}}{m_{0}+\eta_{3}}\right)\left(t-\left(\left(n-1\right)T+lT\right)\right)},\\ \left(n-1\right)T+lT<t\leq nT, \end{array}\right. \end{array}$$

with

(78) $$\begin{array}{c} \left\{\begin{array}{c} {\tilde{z}}^{*}\left(0^{+}\right)=\frac{\left[\left(1-e^{-\left(\delta_{2}-\omega_{2}m_{0}/m_{0}+\eta_{3}\right)\left(1-l\right)T}\right)+\left(1-p_{H}\right)\left(e^{-\left(\delta_{2}-\omega_{2}m_{0}/m_{0}+\eta_{3}\right)\left(1-l\right)T}-e^{-\left(\delta_{2}-\omega_{2}m_{0}/m_{0}+\eta_{3}\right)T}\right)\right]\left(\sigma_{2}/\delta_{2}-\omega_{2}m_{0}/m_{0}+\eta_{3}\right)}{1-\left(1-p_{H}\right)e^{-\left(\delta_{2}-\omega_{2}m_{0}/m_{0}+\eta_{3}\right)T}},\\ {\tilde{z}}^{*}\left(lT^{+}\right)=\left(1-p_{H}\right)\left(\frac{\sigma_{2}}{\delta_{2}-\omega_{2}m_{0}/m_{0}+\eta_{3}}+\left({\tilde{z}}^{*}\left(0^{+}\right)-\frac{\sigma_{2}}{\delta_{2}-\omega_{2}m_{0}/m_{0}+\eta_{3}}\right)e^{-\left(\delta_{2}-\frac{\omega_{2}m_{0}}{m_{0}+\eta_{3}}\right)lT}\right). \end{array}\right. \end{array}$$

Therefore, there exists a *t*_5_ > 0 such that when *t* > *t*_5_, it holds that

(79) $$\begin{array}{c} z\left(t\right)\leq \tilde{z}\left(t\right)<{\tilde{z}}^{*}\left(t\right)+\varepsilon_{5}. \end{array}$$

We show that *x*(*t*) < *m*_0_ cannot hold for all *t* > *t*_5_. In contrast, assume that *x*(*t*) < *m*_0_ holds for all *t* > *t*_5_. Then, consider the following system:

(80) $$\begin{array}{c} \left\{\begin{array}{cc} \frac{dy}{dt}=y\left(\left(\rho \varepsilon_{5}-\delta_{1}\right)+\rho {\tilde{z}}^{*}\left(t\right)\right), & t\neq \left(n-1\right)T+lT,t\neq nT,\\ y\left(t^{+}\right)=\left(1-p_{E}\right)y\left(t\right), & t=\left(n-1\right)T+lT,\\ y\left(t^{+}\right)=y\left(t\right)+\sigma_{1}, & t=nT. \end{array}\right. \end{array}$$

For *t* > *t*_5_, we obtain the following positive periodic solution:

(81) $$\begin{array}{c} {\tilde{y}}^{*}\left(t\right)=\left\{\begin{array}{c} {\tilde{y}}^{*}\left(0^{+}\right)e^{\int_{\left(n-1\right)T^{+}}^{t}\left(\left(\rho \varepsilon_{5}-\delta_{1}\right)+\rho {\tilde{z}}^{*}\left(s\right)\right)ds},\\ \left(n-1\right)T<t\leq \left(n-1\right)T+lT,\\ {\tilde{y}}^{*}\left(lT^{+}\right)e^{\int_{{\left(\left(n-1\right)T+lT\right)}^{+}}^{t}\left(\left(\rho \varepsilon_{5}-\delta_{1}\right)+\rho {\tilde{z}}^{*}\left(s\right)\right)ds},\\ \left(n-1\right)T+lT<t\leq nT, \end{array}\right. \end{array}$$

with

(82) $$\begin{array}{c} \left\{\begin{array}{c} {\tilde{y}}^{*}\left(0^{+}\right)=\frac{\sigma_{1}}{1-\left(1-p_{E}\right)e^{\int_{0^{+}}^{T}\left(\left(\rho \varepsilon_{5}-\delta_{1}\right)+\rho {\tilde{z}}^{*}\left(t\right)\right)dt}},\\ {\tilde{y}}^{*}\left(lT^{+}\right)=\left(1-p_{E}\right){\tilde{y}}^{*}\left(0^{+}\right)e^{\int_{0^{+}}^{lT}\left(\left(\rho \varepsilon_{5}-\delta_{1}\right)+\rho {\tilde{z}}^{*}\left(t\right)\right)dt}. \end{array}\right. \end{array}$$

Similar to Lemma 3, we can prove that $\underset{t⟶+\infty }{\lim}\left(\tilde{y}\left(t\right)-{\tilde{y}}^{*}\left(t\right)\right)=0$, where $\tilde{y}\left(t\right)$ is the solution of (80). Thus, based on (79) and (3), there exists a *t*′_5_ > *t*_5_ such that

(83) $$\begin{array}{c} y\left(t\right)\leq \tilde{y}\left(t\right)<{\tilde{y}}^{*}\left(t\right)+\varepsilon_{5},\text{for }t>t\prime_{5}, \end{array}$$

which implies that

(84) $$\begin{array}{c} \left\{\begin{array}{cc} \frac{dx}{dt}\geq x\left(\alpha -\alpha \beta m_{0}-\frac{{\tilde{y}}^{*}\left(t\right)+\varepsilon_{5}}{\eta_{1}}\right), & t\neq \left(n-1\right)T+lT,t\neq nT,\\ x\left(t^{+}\right)=\left(1-p_{T}\right)x\left(t\right), & t=\left(n-1\right)T+lT,\\ x\left(t^{+}\right)=x\left(t\right), & t=nT, \end{array}\right. \end{array}$$

for *t* > *t*′_5_.

The article "Dynamics of an Antitumour Model with Pulsed Radioimmunotherapy" was published in 2022. Journal: Comput Math Methods Med.

Let *N*_5_ ∈ *Z*_+_ such that (*N*_5_ − 1)*T* + *lT* ≥ *t*′_5_. By integrating (84) on ((*n* − 1)*T* + *lT*, *nT* + *lT*], where *n* ≥ *N*_5_, we obtain

(85) $$\begin{array}{c} x\left({\left(nT+lT\right)}^{+}\right)\geq x\left({\left(\left(n-1\right)T+lT\right)}^{+}\right)\eta \left(m_{0},\varepsilon_{5}\right). \end{array}$$

Then, based on (85) and (74), we have that *x*(((*N*_5_ − 1) + *lT* + *nT*)^+^) ≥ *x*(((*N*_5_ − 1)*T* + *lT*)^+^)(*η*(*m*_0_, *ε*_5_))^*n*^⟶+∞ as *n*⟶∞, which contradicts the boundedness of *x*(*t*). Thus, there exists a *t*_6_ > *t*_5_ > 0 such that *x*(*t*_6_) ≥ *m*_0_.

**Step 2 .**

If *x*(*t*) ≥ *m*_0_ for all *t* ≥ *t*_6_, then our goal is obtained. Otherwise, *x*(*t*) < *m*_0_ for some *t* > *t*_6_. We set *t*^∗^ = inf{*t*|*t* > *t*_6_, *x*(*t*) < *m*_0_}; then, we have *t*^∗^ ≥ *t*_6_ > *t*_5_ > 0, which implies that (45) holds on the interval [*t*^∗^, +∞). Thus, we can consider the following two cases for *t*^∗^:

**Case 1 .**

There exists an *n*_1_ ∈ *Z*_+_ such that *t*^∗^ = *n*_1_*T* + *lT*.

According to the definition of the infimum *t*^∗^ = inf{*t*|*t* > *t*_6_, *x*(*t*) < *m*_0_}, we know that *x*(*t*) ≥ *m*_0_ holds for all *t* ∈ [*t*_6_, *t*^∗^] and *x*(*t*^∗^^+^) ≤ *m*_0_.

We choose *n*_2_, *n*_3_ ∈ *Z*_+_ such that

(86) $$\begin{array}{c} \left\{\begin{array}{c} n_{2}>\frac{\ln\left(\varepsilon_{5}/\left(M_{E}e^{\rho \int_{0^{+}}^{T}{\tilde{z}}^{*}\left(t\right)dt}\right)\right)}{\ln\left(\left(1-p_{E}\right)e^{\int_{0^{+}}^{T}\left(\left(\rho \varepsilon_{5}-\delta_{1}\right)+\rho {\tilde{z}}^{*}\left(t\right)\right)dt}\right)},\\ {\left(1-p_{T}\right)}^{n_{2}}e^{\left(n_{2}+1\right)\overset{\wedge }{\eta }T}{\left(\eta \left(m_{0},\varepsilon_{5}\right)\right)}^{n_{3}}>1, \end{array}\right. \end{array}$$

where $\hat{\eta }=\alpha -\alpha \beta m_{0}-\max\left\{M_{E},\alpha \eta_{1}\right\}/\eta_{1}<0$.

We claim that there exists a *t*_7_ ∈ (*t*^∗^, *t*^∗^ + (*n*_2_ + *n*_3_)*T*) such that *x*(*t*_7_) > *m*_0_. Otherwise, we can assume that *x*(*t*) ≤ *m*_0_ is valid for *t* ∈ (*t*^∗^, *t*^∗^ + (*n*_2_ + *n*_3_)*T*]. Then, similar to Lemma 3, when *t* ∈ (*t*^∗^, *t*^∗^ + (*n*_2_ + *n*_3_)*T*], it holds that

(87) $$\begin{array}{c} \tilde{y}\left(t\right)=\left\{\begin{array}{c} \tilde{y}\left(\left(n-1\right)T^{+}\right)e^{\int_{\left(n-1\right)T^{+}}^{t}\left(\left(\rho \varepsilon_{5}-\delta_{1}\right)+\rho {\tilde{z}}^{*}\left(s\right)\right)ds},\\ \left(n-1\right)T<t\leq \left(n-1\right)T+lT,\\ \tilde{y}\left({\left(\left(n-1\right)T+lT\right)}^{+}\right)e^{\int_{{\left(\left(n-1\right)T+lT\right)}^{+}}^{t}\left(\left(\rho \varepsilon_{5}-\delta_{1}\right)+\rho {\tilde{z}}^{*}\left(s\right)\right)ds},\\ \left(n-1\right)T+lT<t\leq nT, \end{array}\right. \end{array}$$

where $\tilde{y}\left(t\right)$ is the solution of (80). Thus, we obtain

(88) $$\begin{array}{c} \tilde{y}\left({\left(nT+lT\right)}^{+}\right)-{\tilde{y}}^{*}\left({\left(nT+lT\right)}^{+}\right)={\left(\left(1-p_{E}\right)e^{\int_{0^{+}}^{T}\left(\left(\rho \varepsilon_{5}-\delta_{1}\right)+\rho {\tilde{z}}^{*}\left(t\right)\right)dt}\right)}^{n-n_{1}}\times \left(\tilde{y}\left({t^{*}}^{+}\right)-{\tilde{y}}^{*}\left({t^{*}}^{+}\right)\right). \end{array}$$

Then, when *t* ∈ (*t*^∗^ + *n*_2_*T*, *t*^∗^ + (*n*_2_ + *n*_3_)*T*], it follows from (87), (81), (88), (74), and (86) that

(89) $$\begin{array}{c} \tilde{y}\left(t\right)-{\tilde{y}}^{*}\left(t\right)\leq y\left({t^{*}}^{+}\right){\left(\left(1-p_{E}\right)e^{\int_{0^{+}}^{T}\left(\left(\rho \varepsilon_{5}-\delta_{1}\right)+\rho {\tilde{z}}^{*}\left(t\right)\right)dt}\right)}^{n_{2}}\times e^{\rho \int_{0^{+}}^{T}{\tilde{z}}^{*}\left(t\right)dt}<\varepsilon_{5}, \end{array}$$

which implies that

(90) $$\begin{array}{c} y\left(t\right)\leq \tilde{y}\left(t\right)<{\tilde{y}}^{*}\left(t\right)+\varepsilon_{5}, \end{array}$$

for *t* ∈ (*t*^∗^ + *n*_2_*T*, *t*^∗^ + (*n*_2_ + *n*_3_)*T*]. Similar to (85), we have

(91) $$\begin{array}{c} x\left(t^{*}+\left(n_{2}+n_{3}\right)T\right)\geq x\left(t^{*}+n_{2}T\right){\left(\eta \left(m_{0},\varepsilon_{5}\right)\right)}^{n_{3}}. \end{array}$$

On the other hand, in the interval (*t*^∗^, *t*^∗^ + *n*_2_*T*], the following is valid:

(92) $$\begin{array}{c} \left\{\begin{array}{cc} \frac{dx}{dt}\geq x\left(t\right)\hat{\eta }, & t\neq \left(n-1\right)T+lT,t\neq nT,\\ x\left(t^{+}\right)=\left(1-p_{T}\right)x\left(t\right), & t=\left(n-1\right)T+lT,\\ x\left(t^{+}\right)=x\left(t\right), & t=nT, \end{array}\right. \end{array}$$

since *x*(*t*) ≤ *m*_0_ and *y*(*t*) < *M*_*E*_ hold for *t* ∈ (*t*^∗^, *t*^∗^ + *n*_2_*T*]. Integrating (92) on the interval (*t*^∗^, *t*^∗^ + *n*_2_*T*] yields the following:

(93) $$\begin{array}{c} x\left(t^{*}+n_{2}T\right)\geq x\left(t^{*}\right){\left(\left(1-p_{T}\right)e^{\overset{\wedge }{\eta }T}\right)}^{n_{2}}\geq {\left(1-p_{T}\right)}^{n_{2}}m_{0}e^{n_{2}\overset{\wedge }{\eta }T}. \end{array}$$

It follows from (91), (93), and (86) that

(94) $$\begin{array}{c} x\left(t^{*}+\left(n_{2}+n_{3}\right)T\right)>m_{0}, \end{array}$$

which is a contradiction.

The article "Dynamics of an Antitumour Model with Pulsed Radioimmunotherapy" was published in 2022. Journal: Comput Math Methods Med.

Let *t*^∗∗^ = inf{*t*|*t* > *t*^∗^, *x*(*t*) > *m*_0_}; then, *t*^∗∗^ ∈ [*t*^∗^, *t*^∗^ + (*n*_2_ + *n*_3_)*T*), and *x*(*t*) ≤ *m*_0_ holds for *t* ∈ (*t*^∗^, *t*^∗∗^]. Suppose that there exists an *n*_4_ ∈ *Z*_+_ such that *t*^∗∗^ = *n*_4_*T* + *lT*; then, according to *x*(*t*^∗∗^^+^) < *m*_0_, there exists a *δ*_0_ > 0 such that when *t* ∈ (*t*^∗∗^, *t*^∗∗^ + *δ*_0_), *x*(*t*) < *m*_0_ holds, which contradicts the definition of the infimum *t*^∗∗^ = inf{*t*|*t* > *t*^∗^, *x*(*t*) > *m*_0_}. Thus, there is no *n*_4_ ∈ *Z*_+_ such that *t*^∗∗^ = *n*_4_*T* + *lT*. Since *x*(*t*) is continuous at *t* = *t*^∗∗^, we thus have that *x*(*t*^∗∗^) = *m*_0_.

For *t* ∈ (*t*^∗^, *t*^∗∗^), assume that *t*^∗^ + (*n*_5_ − 1)*T* < *t* ≤ *t*^∗^ + *n*_5_*T*, where *n*_5_ ∈ {1, 2, ⋯, *n*_2_ + *n*_3_}. Then, similar to (93), we have that

(95) $$\begin{array}{c} x\left(t\right)\geq {\left(1-p_{T}\right)}^{n_{5}}x\left(t^{*}\right)e^{\left(t-t^{*}\right)\overset{\wedge }{\eta }}\geq m_{1}, \end{array}$$

where

(96) $$\begin{array}{c} m_{1}={\left(1-p_{T}\right)}^{n_{2}+n_{3}}m_{0}e^{\left(n_{2}+n_{3}\right)\overset{\wedge }{\eta }T}. \end{array}$$

For *t* > *t*^∗∗^, the same arguments can be continued since *x*(*t*^∗∗^) = *m*_0_.

The article "Dynamics of an Antitumour Model with Pulsed Radioimmunotherapy" was published in 2022. Journal: Comput Math Methods Med.

**Case 2 .**

There exists no *n* ∈ *Z*_+_ such that *t*^∗^ = *nT* + *lT*.

It is clear that *x*(*t*) ≥ *m*_0_ for *t* ∈ [*t*_6_, *t*^∗^] and *x*(*t*^∗^) = *m*_0_. Suppose that *t*^∗^ ∈ ((*n*_6_ − 1)*T* + *lT*, *n*_6_*T* + *lT*), where *n*_6_ ∈ *Z*_+_.

**Case 3 .**

There exists some *t* ∈ (*t*^∗^, *n*_6_*T* + *lT*) such that *x*(*t*) > *m*_0_.

Let *t*^∗∗∗^ = inf{*t*|*t* > *t*^∗^, *x*(*t*) > *m*_0_}; then, *t*^∗∗∗^ ∈ [*t*^∗^, *n*_6_*T* + *lT*). For *t* ∈ (*t*^∗^, *t*^∗∗∗^), it follows that *x*(*t*) ≤ *m*_0_; thus, *x*(*t*^∗∗∗^) = *m*_0_. Similar to (93), when *t* ∈ (*t*^∗^, *t*^∗∗∗^), we have

(97) $$\begin{array}{c} x\left(t\right)\geq x\left(t^{*}\right)e^{\overset{\wedge }{\eta }\left(t-t^{*}\right)}\geq m_{2}, \end{array}$$

where

(98) $$\begin{array}{c} m_{2}=m_{0}e^{\overset{\wedge }{\eta }T}. \end{array}$$

For *t* > *t*^∗∗∗^, the same arguments can be continued since *x*(*t*^∗∗∗^) = *m*_0_.

**Case 4 .**

For all *t* ∈ (*t*^∗^, *n*_6_*T* + *lT*), *x*(*t*) ≤ *m*_0_.

Let *t*^∗∗∗∗^ = inf{*t*|*t* > *t*^∗^, *x*(*t*) > *m*_0_} ; then, *t*^∗∗∗∗^ ∈ [*n*_6_*T* + *lT*, (*n*_6_*T* + *lT*) + (*n*_2_ + *n*_3_)*T*) and *x*(*t*^∗∗∗∗^^+^) = *m*_0_. Similar to Cases 1 and 3, we can prove that when *t* ∈ (*t*^∗^, *t*^∗∗∗∗^), it holds that

(99) $$\begin{array}{c} x\left(t\right)\geq m_{T}, \end{array}$$

where

(100) $$\begin{array}{c} m_{T}={\left(1-p_{T}\right)}^{n_{2}+n_{3}}m_{0}e^{\left(n_{2}+n_{3}+1\right)\overset{\wedge }{\eta }T}, \end{array}$$

where *m*_*T*_ < *m*_1_ < *m*_2_ < *m*_0_.

We repeat the above procedure to prove that *x*(*t*) ≥ *m*_*T*_ for *t* ≥ *t*_6_.

Furthermore, according to Schauder's fixed point theorem, there exists a tumour-present periodic solution for system (3).

This completes the proof.

## 5. Numerical Analysis

We are interested in how the key factors (i.e., the killing rates *p*_*E*_, *p*_*H*_, and *p*_*T*_, the dosage of infusing the *ECs* (*σ*_1_), the therapeutic period *T*, and the activation rate of the *ECs* (*ρ*)) affect the threshold value *R*_0_ defined in (46). Since ∫_0^+^_^*T*^*y*^∗^(*t*)*dt* is independent of *p*_*T*_, *R*_0_ decreases monotonically with respect to *p*_*T*_, indicating that the strong tumour cell killing effect of radiotherapy can increase tumour cell death.

First, we set the parameters as follows [16, 17]:

(101) $$\begin{array}{c} \begin{array}{ccc} \delta_{1}=0.3473, & \sigma_{2}=0.38, & \delta_{2}=0.055,\\ \omega_{2}=0.02, & \eta_{3}=0.1, & \alpha =1.636,\\ \eta_{1}=0.1, & l=0.5. & \;. \end{array} \end{array}$$

Figure 3(a) shows that when *p*_*H*_ (or *p*_*E*_) decreases to the threshold value *T*_*p*_*H*__ = 0.1440 (or *T*_*p*_*E*__ = 0.0377) of the tumour-free periodic solution, *R*_0_ monotonically decreases to 0. In addition, when *T*_*p*_*H*__ < *p*_*E*_, *p*_*H*_ < 0.2, *R*_0_(*p*_*H*_) is much smaller than *R*_0_(*p*_*E*_), where *R*_0_(*p*_*E*_) > 1. Therefore, in this case, the optimal control strategy is achieved when *p*_*H*_ and *p*_*E*_ are sufficiently small, and, compared to parameter *p*_*E*_, a smaller parameter *p*_*H*_ is more beneficial for tumour control. Similarly, Figures 3(b) and 3(c) show that *R*_0_ monotonically decreases as *σ*_1_ increases or *T* decreases, indicating that a higher dosage of infusing the *ECs* or more frequent radioimmunotherapy can accelerate the eradication of tumour cells. In addition, Figure 3(d) shows that when *ρ* increases to the threshold value *T*_*ρ*_ = 0.2003 of the tumour-free periodic solution, *R*_0_ rapidly decreases to 0. Thus, strong activation of the *ECs* by the *HTCs* is beneficial for tumour control.

The article "Dynamics of an Antitumour Model with Pulsed Radioimmunotherapy" was published in 2022. Journal: Comput Math Methods Med.

Moreover, when *σ*_1_ = 0 and

(102) $$\begin{array}{c} R_{0}=\left(1-p_{T}\right)e^{\alpha T}>1, \end{array}$$

it follows from Theorem 5 (i) that the tumour-free periodic solution is unstable for radiotherapy alone. For example, if we fix the parameters as those shown in Figures 1(a)–1(c), the tumour cell population oscillates as a periodic cycle. Similar results are observed for the case of immunotherapy alone (see Figures 1(d)–1(f)). On the other hand, if we set the parameter values as those shown in Figures 4(a)–4(c), the tumour cells are eventually eradicated with radioimmunotherapy. Thus, we can say that radioimmunotherapy is more effective than therapy regimes with radiotherapy or immunotherapy alone.

Furthermore, Figure 5 displays bifurcation diagrams for system (3). The dynamical behaviour of system (3) is dominated by tumour-free and tumour-present periodic solutions. When *T* is smaller than the threshold value *T*_*a*_ = 2.0076, the global attractiveness of the tumour-free periodic solution can be validated (see Figures 4(a)–4(c)). However, when *T*_*a*_ < *T* < *T*_*p*_ = 5.733, where *T*_*p*_ is the threshold value for the permanence of system (3), the emergence of a tumour-present periodic solution leads to the local stability of the tumour-free periodic solution (see Figures 4(d)–4(f) and Figures 2(a)–2(c)). In addition, when *T* > *T*_*p*_ = 5.733, all three cell populations oscillate periodically, which indicates that system (3) is permanent and has a tumour-present periodic solution (see Figures 2(d)–2(f)). In particular, the complex patterns shown in Figures 2, 4, and 5 demonstrate that a properly designed control period *T* is crucial for successful tumour control.

The article "Dynamics of an Antitumour Model with Pulsed Radioimmunotherapy" was published in 2022. Journal: Comput Math Methods Med.

## 6. Discussion

In this paper, we develop a tumour-immune model with pulsed treatments to show how radiotherapy and immunotherapy affect the dynamics of tumour treatments. It is assumed that the radiotherapy and immunotherapy are administered with the same periodicity but not simultaneously. Additionally, it is assumed that fixed proportions of tumour cells, effector cells, and helper T cells are degraded each time the radiotherapy is administered.

Similar to the proof of the continuity of the solution with respect to the right-hand side of the ordinary differential equations, we proved that $\underset{t⟶+\infty }{\lim}\left|y\left(t\right)-y^{*}\left(t\right)\right|=0$ in Lemma 3 by using the integral inequality technique. Then, based on the differentiability of the solution with respect to the initial values, we determined the eigenvalues of the Jacobian matrix at the fixed point corresponding to the tumour-free periodic solution, which was used to obtain the local stability threshold condition. Furthermore, the indicator *R*_0_ is provided as a sufficient condition for the global attractiveness of the tumour-free periodic solution. We emphasize that a comparison of the solutions of the ordinary differential equations is critical for proving this claim. Biologically speaking, (46) indicates that the tumour cells have been completely eradicated throughout the body, indicating the ultimate success of our treatment strategy. Similarly, we proved that system (3) is permanent with at least one tumour-present periodic solution under certain conditions, suggesting that tumour cells, effector cells, and helper T cells coexist indefinitely in the tumour-present periodic solution. It is clear that *t* = *t*_5_ is an important threshold value for our proof since $z\left(t\right)<{\overset{\sim }{z}}^{***}\left(t\right)+\varepsilon_{5}$ for *t* > *t*_5_.

Our results demonstrate that the effectiveness of radioimmunotherapy, the therapeutic period, and the activation rate of the *ECs* by the *HTCs* are all crucial for tumour depression and resurgence. The numerical results presented in Section 5 indicate that *R*_0_ is sensitive to small changes in the killing rates *p*_*E*_, *p*_*H*_, and *p*_*T*_, the dosage *σ*_1_ of infusing the *ECs*, the therapeutic period *T*, and the activation rate *ρ* of the *ECs*; that is, the smaller (or larger) the parameters *p*_*E*_, *p*_*H*_, and *T* (or *p*_*T*_, *σ*_1_, and *ρ*) are, the smaller the indicator *R*_0_ is. In particular, decreases in *p*_*H*_ are more beneficial for tumour control than decreases in *p*_*E*_, and radioimmunotherapy is more effective than either radiotherapy or immunotherapy alone.

The article "Dynamics of an Antitumour Model with Pulsed Radioimmunotherapy" was published in 2022. Journal: Comput Math Methods Med.

Furthermore, we performed one-parameter bifurcation analyses on the threshold value *R*_0_, as shown in Figure 5. Figure 5 shows the impact of the period *T* on the threshold value *R*_0_. The tumour-free periodic solution is locally stable for *T*_*a*_ < *T* < *T*_*p*_, whereas system (3) is permanent with a tumour-present periodic solution for *T* > *T*_*p*_.  Figure 2 shows that if *T* is increased from 5 to 6, the permanence of system (3) causes the tumour-free periodic solution to lose its local stability. These results demonstrate that the parameters *p*_*E*_, *p*_*H*_, *p*_*T*_, *σ*_1_, *T*, and *ρ* are crucial for tumour control. This information may help doctors in designing and determining the optimum therapeutic approaches for tumour control.

As a comparison to other relevant studies, we note the following highlights of our study: (i) note that system (3) in [24] includes only one impulsive control strategy (injecting the effector cells into the body), while system (4) in [24] and system (1) in [27] include only the tumour cells and effector cells. However, system (3) includes not only helper T cells but also two impulsive control strategies that are not implemented simultaneously. (ii) In contrast to the small amplitude perturbation method used in [24], we use a more rigorous method to prove the local stability of the tumour-free periodic solution of system (2) with. (iii) Although the proofs of the permanence of the corresponding impulsive systems in [24, 27] are omitted, we include the proof of the permanence of our system in this study.

Similar to [28, 29], the existence of tumour-present periodic solutions for system (3) was investigated in our study. Furthermore, based on the techniques used in [30–34], we hypothesize that the existence and global attractiveness of the tumour-present periodic solution of system (3) can be proven by using Lyapunov's second method. This proof will be demonstrated in our future research.

## Figures and Tables

**Figure 1:** Dynamic behaviours of system (3) with radiotherapy or immunotherapy alone. (a)–(c) *ρ* = 0.01, *β* = 0.002, *p*_*E*_ = 0.15, *p*_*H*_ = 0.1, *p*_*T*_ = 0.9619, *σ*_1_ = 0, and *T* = 2; (d)–(f): *ρ* = 0.01, *β* = 0.002, *p*_*E*_ = 0, *p*_*H*_ = 0, *p*_*T*_ = 0, *σ*_1_ = 2, and *T* = 2. The other parameters are identical to those in (101), and the initial values in (a)–(f) are (1, 1, 500).

**Figure 2:** Dynamic behaviours of system (3), where *T* = 5 in (a)–(c) and *T* = 6 in (d)–(f). The other parameters are identical to those in Figure 5, and the initial values in (a)–(f) are (0.2442,5.0060,0.0256).

**Figure 3:** Simulations of the effects of *p*_*E*_, *p*_*H*_, *σ*_1_, *T*, and *ρ* on *R*_0_. The baseline parameters are *ρ* = 0.16, *β* = 0.3, *p*_*E*_ = 0.2, *p*_*H*_ = 0.2, *p*_*T*_ = 0.85, *σ*_1_ = 0.2, and *T* = 2, and the other relevant parameters are identical to those in (101).

The article "Dynamics of an Antitumour Model with Pulsed Radioimmunotherapy" was published in 2022. Journal: Comput Math Methods Med.

**Figure 4:** Dynamic behaviours of system (2) with radioimmunotherapy. (a)–(c) *ρ* = 0.01, *β* = 0.002, *p*_*E*_ = 0.15, *p*_*H*_ = 0.1, *p*_*T*_ = 0.9619, *σ*_1_ = 2, and *T* = 2; (d)–(f) *ρ* = 0.01, *β* = 0.002, *p*_*E*_ = 0.2, *p*_*H*_ = 0.1, *p*_*T*_ = 0.9625, *σ*_1_ = 0.2, and *T* = 5. The other parameters are identical to those in (101), and the initial values in (a)–(f) are (1, 1, 500).

**Figure 5:** Bifurcation diagrams for system (3) with respect to *T*, where *ρ* = 0.01, *β* = 0.002, *p*_*E*_ = 0.2, *p*_*H*_ = 0.1, *p*_*T*_ = 0.9625, and *σ*_1_ = 0.2. The other parameters are identical to those in (101).

## Data Availability

There is no underlying data supporting the results of our study.

## Appendix

### A. The Jacobian Matrix of Map Ψ(*X*^0^) at Point *X*_0_ = (*y*_0_, *z*_0_, 0)

Denote

(A.1) $$\begin{array}{c} F\left(X\right)={\left(-\delta_{1}y+\rho yz,\sigma_{2}-\delta_{2}z+\omega_{2}z\frac{x}{x+\eta_{3}},\alpha x\left(1-\beta x\right)-y\frac{x}{x+\eta_{1}}\right)}^{T}, \end{array}$$

where *X* = (*y*, *z*, *x*). Based on the differentiability of the solution with respect to the initial values, we obtain

(A.2) $$\begin{array}{c} \frac{d}{dt}\left[D_{X^{0}}\Phi \left(t;t_{0},X^{0}\right)\right]=D_{X}F\left(\Phi \left(t;t_{0},X^{0}\right)\right)D_{X^{0}}\Phi \left(t;t_{0},X^{0}\right). \end{array}$$

Specifically, when *X*^0^ = (*y*_0_, *z*_0_, 0)≜*X*_0_, we have

(A.3) $$\begin{array}{c} \frac{d}{dt}\left[D_{X^{0}}\Phi \left(t;t_{0},X_{0}\right)\right]=D_{X}F\left(\Phi \left(t;t_{0},X_{0}\right)\right)D_{X^{0}}\Phi \left(t;t_{0},X_{0}\right). \end{array}$$

According to the first three equations of (3), it is clear that

(A.4) $$\begin{array}{c} \Phi \left(t;t_{0},X_{0}\right)=\left(y\left(t;t_{0},X_{0}\right),z\left(t;t_{0},X_{0}\right),0\right),\text{for }t\geq t_{0}; \end{array}$$

thus,

(A.5) $$\begin{array}{c} \left\{\begin{array}{c} \frac{\partial x\left(t;t_{0},X_{0}\right)=0,}{\partial y^{0}}\\ \frac{\partial x\left(t;t_{0},X_{0}\right)}{\partial z^{0}}=0, \end{array}\right. \end{array}$$

for *t* ≥ *t*_0_. In addition, it follows from (A.1) that

(A.6) $$\begin{array}{c} D_{X}F\left(X\right)=\left(\begin{array}{ccc} -\delta_{1}+\rho z & \rho y & 0\\ 0 & -\delta_{2}+\omega_{2}\frac{x}{x+\eta_{3}} & \omega_{2}z\frac{\eta_{3}}{{\left(x+\eta_{3}\right)}^{2}}\\ -\frac{x}{x+\eta_{1}} & 0 & \alpha \left(1-2\beta x\right)-y\frac{\eta_{1}}{{\left(x+\eta_{1}\right)}^{2}} \end{array}\right). \end{array}$$

Substituting (A.6), (A.4), and (A.5) into (A.3) yields

(A.7) $$\begin{array}{c} \frac{d}{dt}\left(\begin{array}{ccc} \frac{\partial y}{\partial y^{0}} & \frac{\partial y}{\partial z^{0}} & \frac{\partial y}{\partial x^{0}}\\ \frac{\partial z}{\partial y^{0}} & \frac{\partial z}{\partial z^{0}} & \frac{\partial z}{\partial x^{0}}\\ 0 & 0 & \frac{\partial x}{\partial x^{0}} \end{array}\right)\left(t;t_{0},X_{0}\right)=\left(\begin{array}{ccc} -\delta_{1}+\rho z\left(t;t_{0},X_{0}\right) & \rho y\left(t;t_{0},X_{0}\right) & 0\\ 0 & -\delta_{2} & \frac{\omega_{2}z\left(t;t_{0},X_{0}\right)}{\eta_{3}}\\ 0 & 0 & \alpha -\frac{y\left(t;t_{0},X_{0}\right)}{\eta_{1}} \end{array}\right)\times \left(\begin{array}{ccc} \frac{\partial y}{\partial y^{0}} & \frac{\partial y}{\partial z^{0}} & \frac{\partial y}{\partial x^{0}}\\ \frac{\partial z}{\partial y^{0}} & \frac{\partial z}{\partial z^{0}} & \frac{\partial z}{\partial x^{0}}\\ 0 & 0 & \frac{\partial x}{\partial x^{0}} \end{array}\right)\left(t;t_{0},X_{0}\right), \end{array}$$

which implies that

(A.8) $$\begin{array}{c} \left\{\begin{array}{c} \frac{d}{dt}\left(\frac{\partial y}{\partial y^{0}}\left(t;t_{0},X_{0}\right)\right)=\left(-\delta_{1}+\rho z\left(t;t_{0},X_{0}\right)\right)\frac{\partial y}{\partial y^{0}}\left(t;t_{0},X_{0}\right)+\rho y\left(t;t_{0},X_{0}\right)\frac{\partial z}{\partial y^{0}}\left(t;t_{0},X_{0}\right),\\ \frac{d}{dt}\left(\frac{\partial z}{\partial y^{0}}\left(t;t_{0},X_{0}\right)\right)--\delta_{2}\frac{\partial z}{\partial y^{0}}\left(t;t_{0},X_{0}\right),\\ \begin{array}{c} \frac{d}{dt}\left(\frac{\partial z}{\partial z^{0}}\left(t;t_{0},X_{0}\right)\right)=-\delta_{2}\frac{\partial z}{\partial z^{0}}\left(t;t_{0},X_{0}\right),\\ \frac{d}{dt}\left(\frac{\partial x}{\partial x^{0}}\left(t;t_{0},X_{0}\right)\right)=\left(\alpha -\frac{y\left(t;t_{0},X_{0}\right)}{\eta_{1}}\right)\frac{\partial x}{\partial x^{0}}\left(t;t_{0},X_{0}\right),\\ \begin{array}{c} \frac{\partial y}{\partial y^{0}}\left(t_{0};t_{0},X_{0}\right)=1,\\ \begin{array}{c} \frac{\partial z}{\partial y^{0}}\left(t_{0};t_{0},X_{0}\right)=0,\\ \frac{\partial z}{\partial z^{0}}\left(t_{0};t_{0},X_{0}\right)=1,\\ \frac{\partial x}{\partial x^{0}}\left(t_{0};t_{0},X_{0}\right)=1. \end{array} \end{array} \end{array} \end{array}\right. \end{array}$$

Solving (A.8) yields

(A.9) $$\begin{array}{c} \left\{\begin{array}{c} \frac{\partial y}{\partial y^{0}}\left(t;t_{0},X_{0}\right)=e^{\int_{t_{0}}^{t}\left(-\delta_{1}+\rho z\left(s;t_{0},X_{0}\right)\right)ds},\\ \frac{\partial z}{\partial y^{0}}\left(t;t_{0},X_{0}\right)=0,\\ \frac{\partial z}{\partial z^{0}}\left(t;t_{0},X_{0}\right)=e^{-\delta_{2}\left(t-t_{0}\right)},\\ \frac{\partial x}{\partial x^{0}}\left(t;t_{0},X_{0}\right)=e^{\int_{t_{0}}^{t}\left(\alpha -\frac{y\left(s;t_{0},X_{0}\right)}{\eta_{1}}\right)ds}. \end{array}\right. \end{array}$$

According to (A.5) and (A.9), we have

(A.10) $$\begin{array}{c} D_{X^{0}}\Phi \left(t;t_{0},X_{0}\right)=\left(\begin{array}{ccc} \frac{\partial y\left(t;t_{0},X_{0}\right)}{\partial y^{0}} & \frac{\partial y\left(t;t_{0},X_{0}\right)}{\partial z^{0}} & \frac{\partial y\left(t;t_{0},X_{0}\right)}{\partial x^{0}}\\ 0 & \frac{\partial z\left(t;t_{0},X_{0}\right)}{\partial z^{0}} & \frac{\partial z\left(t;t_{0},X_{0}\right)}{\partial x^{0}}\\ 0 & 0 & \frac{\partial x\left(t;t_{0},X_{0}\right)}{\partial x^{0}} \end{array}\right). \end{array}$$

Then, based on (44), (43), (A.10), and (A.9), we obtain

(A.11) $$\begin{array}{c} D_{X^{0}}\Psi \left(X^{0}\right)=D_{X^{0}}\Phi \left(\left(1-l\right)T,I_{1}\left(\Phi \left(lT,X^{0}\right)\right)\right)\times \left(\begin{array}{ccc} 1-p_{E} & 0 & 0\\ 0 & 1-p_{H} & 0\\ 0 & 0 & 1-p_{T} \end{array}\right)D_{X^{0}}\Phi \left(l_{1}T,X^{0}\right). \end{array}$$

Furthermore,

(A.12) $$\begin{array}{c} D_{X^{0}}\Psi \left(X_{0}\right)=\left(\begin{array}{ccc} \frac{\partial y}{\partial y^{0}} & \frac{\partial y}{\partial z^{0}} & \frac{\partial y}{\partial x^{0}}\\ 0 & \frac{\partial z}{\partial z^{0}} & \frac{\partial z}{\partial x^{0}}\\ 0 & 0 & \frac{\partial x}{\partial x^{0}}. \end{array}\right)\left(\left(1-l\right)T,I_{1}\left(\Phi \left(lT,X_{0}\right)\right)\right)\times \left(\begin{array}{ccc} \left(1-p_{E}\right)\frac{\partial y}{\partial y^{0}} & \left(1-p_{E}\right)\frac{\partial y}{\partial z^{0}} & \left(1-p_{E}\right)\frac{\partial y}{\partial x^{0}}\\ 0 & \left(1-p_{H}\right)\frac{\partial z}{\partial z^{0}} & \left(1-p_{H}\right)\frac{\partial z}{\partial x^{0}}\\ 0 & 0 & \left(1-p_{T}\right)\frac{\partial x}{\partial x^{0}}. \end{array}\right)\left(lT,X_{0}\right)≜\left(\begin{array}{ccc} a_{0} & * & *\\ 0 & b_{0} & *\\ 0 & 0 & c_{0} \end{array}\right), \end{array}$$

where

(A.13) $$\begin{array}{c} \left\{\begin{array}{c} a_{0}=\left(1-p_{E}\right)\frac{\partial y\left(\left(1-l\right)T,I_{1}\left(\Phi \left(lT,X_{0}\right)\right)\right)}{\partial y^{0}}\frac{\partial y\left(l_{1}T,X_{0}\right)}{\partial y^{0}}=\left(1-p_{E}\right)\times e^{\int_{0}^{\left(1-l\right)T}\left(-\delta_{1}+\rho z\left(s,I_{1}\left(\Phi \left(lT,X_{0}\right)\right)\right)\right)ds+\int_{0}^{lT}\left(-\delta_{1}+\rho z\left(s,X_{0}\right)\right)ds},\\ b_{0}=\left(1-p_{H}\right)\frac{\partial z\left(\left(1-l\right)T,I_{1}\left(\Phi \left(lT,X_{0}\right)\right)\right)}{\partial z^{0}}\frac{\partial z\left(l_{1}T,X_{0}\right)}{\partial z^{0}}=\left(1-p_{H}\right)e^{-\delta_{2}T}<1,\\ c_{0}=\left(1-p_{T}\right)\frac{\partial x\left(\left(1-l\right)T,I_{1}\left(\Phi \left(lT,X_{0}\right)\right)\right)}{\partial x^{0}}\frac{\partial x\left(l_{1}T,X_{0}\right)}{\partial x^{0}}=\left(1-p_{T}\right)\times e^{\int_{0}^{\left(1-l\right)T}\left(\alpha -\frac{y\left(s,I_{1}\left(\Phi \left(lT,X_{0}\right)\right)\right)}{\eta_{1}}\right)ds+\int_{0}^{lT}\left(\alpha -\frac{y\left(s,X_{0}\right)}{\eta_{1}}\right)ds}. \end{array}\right. \end{array}$$

The article "Dynamics of an Antitumour Model with Pulsed Radioimmunotherapy" was published in 2022. Journal: Comput Math Methods Med.

## References

[1] Who WHO. https://www.who.int/en/news-room/fact-sheets/detail/cancer.

[2] Mamat M., Subiyanto K. A., Kartono A. (2013). Mathematical model of cancer treatments using immunotherapy, chemotherapy and biochemotherapy. *Applied Mathematical Sciences*.

[3] Das P., Das S., Das P., Rihan F. A., Uzuntarla M., Ghosh D. (2021). Optimal control strategy for cancer remission using combinatorial therapy: a mathematical model-based approach. *Chaos, Solitons & Fractals*.

[4] Chamseddine I. M., Rejniak K. A. (2020). Hybrid modeling frameworks of tumor development and treatment. *Wiley Interdisciplinary Reviews: Systems Biology and Medicine*.

[5] Berraondo P., Sanmamed M. F., Ochoa M. C. (2019). Cytokines in clinical cancer immunotherapy. *British Journal of Cancer*.

[6] López Á. G., Iarosz K. C., Batista A. M., Seoane J. M., Viana R. L., Sanjuán M. A. F. (2019). The role of dose density in combination cancer chemotherapy. *Communications in Nonlinear Science and Numerical Simulation*.

[7] López Alfonso J. C., Poleszczuk J., Walker R. (2019). Immunologic consequences of sequencing cancer radiotherapy and surgery. *JCO Clinical Cancer Informatics*.

[8] Abernathy Z., Abernathy K., Stevens J. (2020). A mathematical model for tumor growth and treatment using virotherapy. *AIMS Mathematics*.

[9] Alqudah M. A. (2020). Cancer treatment by stem cells and chemotherapy as a mathematical model with numerical simulations. *Alexandria Engineering Journal*.

[10] Coletti R., Pugliese A., Marchetti L. (2021). Modeling the effect of immunotherapies on human castration-resistant prostate cancer. *Journal of Theoretical Biology*.

[11] Valle P. A., Coria L. N., Carballo K. D. (2021). Chemoimmunotherapy for the treatment of prostate cancer: insights from mathematical modelling. *Applied Mathematical Modelling*.

[12] Antonov A., Nenov S., Tsvetkov T. (2019). Impulsive controlability of tumor growth. *Dynamic Systems and Applications*.

[13] Sigal D., Przedborski M., Sivaloganathan D., Kohandel M. (2019). Mathematical modelling of cancer stem cell-targeted immunotherapy. *Mathematical biosciences*.

[14] Pratap J. An optimal control strategy for mathematically modeling cancer combination therapy. https://arxiv.org/abs/2101.12120v1.

The article "Dynamics of an Antitumour Model with Pulsed Radioimmunotherapy" was published in 2022. Journal: Comput Math Methods Med.

[15] Feng P., Navaratna M. (2021). Role of regulatory T cells on a simple tumor-immune interaction system. *Communications in Nonlinear Science and Numerical Simulation*.

[16] Dong Y., Miyazaki R., Takeuchi Y. (2014). Mathematical modeling on helper T cells in a tumor immune system. *Discrete & Continuous Dynamical Systems-B*.

[17] Talkington A., Dantoin C., Durrett R. (2018). Ordinary differential equation models for adoptive immunotherapy. *Bulletin of Mathematical Biology*.

[18] Pang L., Zhao Z., Liu S., Zhang X. (2017). Dynamic analysis of an antitumor model and investigation of the therapeutic effects for different treatment regimens. *Computational and Applied Mathematics*.

[19] Cruikshank A. (2021). *A Mathematical Model of Pancreatic Cancer Growth and Response to Treatment, [M.S. thesis]*.

[20] González-Crespo I., Gómez-Caamaño A., Pouso Ó. L. A biomathematical model of tumor response to radioimmunotherapy with *α*PDL1 and *α*CTL4. https://arxiv.org/abs/2106.07591.

[21] Darandis N., Nazari M. (2020). *A mathematical model for chemo-immunotherapy of cancer considering macrophages polarization and cytokine dynamics*.

[22] Makhlouf A. M., El-Shennawy L., Elkaranshawy H. A. (2020). Mathematical modelling for the role of CD4^+^ T cells in tumor-immune interactions. *Computational and mathematical methods in medicine*.

[23] Sung W., Grassberger C., McNamara A. L. (2020). A tumor-immune interaction model for hepatocellular carcinoma based on measured lymphocyte counts in patients undergoing radiotherapy. *Radiotherapy and Oncology*.

[24] Wang J., Zhang Y. (2022). Dynamics of immunotherapy antitumor models with impulsive control strategy. *Mathematical Methods in the Applied Sciences*.

[25] Bainov D., Simeonov P. (1993). *Impulsive Differential Equations: Periodic Solutions and Applications*.

[26] Lakshmikantham V., Simeonov P. S. (1989). *Theory of Impulsive Differential Equations*.

[27] Zhao Z., Pang L., Li Q. (2021). Analysis of a hybrid impulsive tumor-immune model with immunotherapy and chemotherapy. *Chaos, Solitons & Fractals*.

[28] Ma X., Shu X. B., Mao J. (2020). Existence of almost periodic solutions for fractional impulsive neutral stochastic differential equations with infinite delay. *Stochastics and Dynamics*.

[29] Guo Y., Shu X. B., Yin Q. (2021). Existence of solutions for first-order Hamiltonian random impulsive differential equations with Dirichlet boundary conditions. *Discrete & Continuous Dynamical Systems-B*.

[30] Tan R., Liu Z., Cheke R. A. (2012). Periodicity and stability in a single-species model governed by impulsive differential equation. *Applied Mathematical Modelling*.

The article "Dynamics of an Antitumour Model with Pulsed Radioimmunotherapy" was published in 2022. Journal: Comput Math Methods Med.

[31] Li X., Bohner M., Wang C. K. (2015). Impulsive differential equations: periodic solutions and applications. *Automatica*.

[32] Tamen A. T., Dumont Y., Tewa J. J., Bowong S., Couteron P. (2017). A minimalistic model of tree–grass interactions using impulsive differential equations and non-linear feedback functions of grass biomass onto fire-induced tree mortality. *Mathematics and Computers in Simulation*.

[33] Lin Q., Xie X., Chen F., Lin Q. (2018). Dynamical analysis of a logistic model with impulsive Holling type-II harvesting. *Advances in Difference Equations*.

[34] Sun L., Zhu H., Ding Y. (2020). Impulsive control for persistence and periodicity of logistic systems. *Mathematics and Computers in Simulation*.

